The article "q-Rung Orthopair Fuzzy Rough Einstein Aggregation Information-Based EDAS Method: Applications in Robotic Agrifarming" was published in 2021. Journal: Comput Intell Neurosci.

# *q*-Rung Orthopair Fuzzy Rough Einstein Aggregation Information-Based EDAS Method: Applications in Robotic Agrifarming

**DOI:** 10.1155/2021/5520264

**Published:** 2021-10-30

**Authors:** Shahzaib Ashraf, Noor Rehman, Azmat Hussain, Hussain AlSalman, Abdu H. Gumaei

**Affiliations:** ^1^Department of Mathematics and Statistics, Bacha Khan University, Charsadda 24420, Khyber Pakhtunkhwa, Pakistan; ^2^Department of Mathematics and Statistics, International Islamic University, Isalambad, Pakistan; ^3^Department of Computer Science, College of Computer and Information Sciences, King Saud University, Riyadh 11543, Saudi Arabia; ^4^Computer Science Department, Faculty of Applied Sciences, Taiz University, Taiz 6803, Yemen

## Abstract

The main purpose of this manuscript is to present a novel idea on the *q*-rung orthopair fuzzy rough set (*q*-ROFRS) by the hybridized notion of *q*-ROFRSs and rough sets (RSs) and discuss its basic operations. Furthermore, by utilizing the developed concept, a list of *q*-ROFR Einstein weighted averaging and geometric aggregation operators are presented which are based on algebraic and Einstein norms. Similarly, some interesting characteristics of these operators are initiated. Moreover, the concept of the entropy and distance measures is presented to utilize the decision makers' unknown weights as well as attributes' weight information. The EDAS (evaluation based on distance from average solution) methodology plays a crucial role in decision-making challenges, especially when the problems of multicriteria group decision-making (MCGDM) include more competing criteria. The core of this study is to develop a decision-making algorithm based on the entropy measure, aggregation information, and EDAS methodology to handle the uncertainty in real-word decision-making problems (DMPs) under *q*-rung orthopair fuzzy rough information. To show the superiority and applicability of the developed technique, a numerical case study of a real-life DMP in agriculture farming is considered. Findings indicate that the suggested decision-making model is much more efficient and reliable to tackle uncertain information based on *q*-ROFR information.

## 1. Introduction

In the history of agriculture, the domestication of plants and animals, as well as the manufacturing and dissemination techniques for cultivating them productively, is documented. Agriculture began independently in several places of the world and included a broad range of taxa. Farming was well known on the Nile's banks by 8000 BC. Around this time, agriculture evolved independently in the Far East, most likely in China, with rice as the primary crop rather than wheat. Overstretched water supplies, high levels of deforestation, and decreased soil fertility have all resulted from modern farming practices. Since there is insufficient water to continue farming as is, how vital water, ground, and environment resources are used to increase crop yields must be reevaluated. Giving ecosystems importance, understanding environmental and livelihood tradeoffs, and balancing the rights of a range of users and interests may be a solution. Inequities that occur as a result of such steps, such as water reallocation from poor to wealthy and land clearing to make room for more profitable farmland, need to be tackled. Technological advances aid in the provision of tools and services to farmers in order to help them become more prosperous. Conservation tillage, a farming technique that helps avoid land loss due to deforestation, reduces water pollution, and improves carbon sequestration, is one example of a technology-enabled innovation.

To meet the growing demand for food, farming, which was never an easy job to begin with, now needs more analytics and technology. In one case, mathematicians, hydrologists, and farmers met in California to formulate a strategy that would reduce the amount of water used for crops while still making a profit for the farmers and satisfying market demand. The mathematical model used data including plant growth properties and water requirements to determine which crops to plant, when to plant them, and which areas should be left unplanted. Farmers were satisfied to wisely use their own and community tools, while mathematicians were happy to collaborate with business experts.

Pawlak [1] initiated the important notion of rough set (RS) theory. The theory of rough set is the general version of classic set theory, handling imprecise and ambiguous data. The idea of fuzzy rough sets (FRSs) was presented by Dubois and Prade [2]. Zhang and Zhan [3] presented the DMPs using FRSs. The concept of probabilistic hesitant FRS was presented by Khan et al. [4]. Mi et al. [5] presented the uncertainty measure using partition under FRSs. Sun and Ma [6] established the soft FRSs and explained their applicability in DMPs. Zhang et al. [7] extended the structure of the FRS to intuitionistic FRSs to facilitate the decision maker to make their decision to tackle uncertain information freely. Chinram et al. [8] presented the EDAS methodology based on intuitionistic FRSs to handle the multiattribute DMPs. Zhou and Wu [9] developed the generalized approximation operators based on intuitionistic FRSs. Liu et al. [10] developed the preference relation-based decision-making methodology under FRSs. Khan et al. [4] developed the idea of the probabilistic hesitant fuzzy rough set and discussed its application in decision-making.

Pythagorean fuzzy sets are the generalization of fuzzy sets (FSs) [11] and intuitionistic FSs [12] to tackle the uncertain information in the form of (*μ*, *ν*), where *μ* represents the positive grade and *ν* represents the negative grade function, with condition that *μ*^2^+*ν*^2^ ≤ 1. Many authors contribute to Pythagorean FSs: Ding and Liu [13] introduced an approach under Pythagorean fuzzy uncertain linguistic information. Fei and Deng [14] presented the decision support model, and Huang et al. [15] introduced the MULTIMOORA method under Pythagorean fuzzy information. Khan et al. [16] established the Dombi operators, and Liu et al. [17] presented the linguistic Muirhead mean operators under Pythagorean fuzzy settings. Rani et al. [18] developed the extended TOPSIS, and Wei and Lu [19] established the power operators under Pythagorean fuzzy data. Zhang [20] proposed the list of similarity measures under Pythagorean fuzzy settings. Batool et al. [21] developed the novel idea of Pythagorean probabilistic hesitant FSs and discussed their applicability in decision-making.

There are countless examples in real-life situations [22–26] when decision makers (DMs) have strong opinions about grading government programs, projects, or political pronouncements. Allow the administration of a university, for example, to begin megaprojects such as a cricket ground in order to demonstrate its accomplishment and performance. Members of the university administration can give their project a high rating by providing DM (*μ*=0.9); people, on the contrary, may view the same effort as a waste of money and attempt to diminish it by presenting opposing opinions. So, they assign DNM (*ν*=0.7). In this situation, *μ*+*ν* > 1 [12] and *μ*^2^+*ν*^2^ > 1 [27], but *μ*^*q*^+*ν*^*q*^ < 1 for *q* ≥ 2 [28] so that (*μ*, *ν*) is neither an intuitionistic fuzzy number nor a Pythagorean fuzzy number, but it is a *q*-rung orthopair fuzzy number (*q*-ROPFN). *q*-ROPFNs [28] are more efficient to handle vagueness in the data. Many authors contribute to *q*-rung orthopair fuzzy sets (*q*-ROPFSs) in many fields such as decision-making, information measures, knowledge measures, distance measures, and aggregation information. Hussain et al. [29] proposed the list of soft average operators, and Peng et al. [30] presented the exponential function-based aggregation operators under *q*-ROPFSs. Joshi and Gegov [31] introduced the algebraic operators using confidence levels under *q*-ROPFSs. The information measures for *q*-ROPFSs were explored by Peng and Liu [32]. Gao et al. [33] introduced the continuities, derivatives, and differentials for *q*-ROPFNs. Khan et al. [34, 35] proposed the knowledge measure for the *q*-ROPFSs and discussed its applicability in DMPs. Liu and Liu [36] developed the Bonferroni mean operators for the *q*-ROPFSs. Khoshaim et al. [37] presented the novel emergency decision-making methodology under *q*-ROPF rough aggregation information and discussed its applicability to tackle the uncertainty in the emergency situation of COVID-19. Riaz et al. [38] introduced the robust *q*-ROPF Einstein aggregation operators. Verma [39] presented the decision-making algorithm based on order-*α* divergence and entropy measures, and Wang et al. [40] presented the MABAC technique for the *q*-ROPFSs.

*q*-ROPF rough sets (*q*-ROPFRSs) are a hybrid intelligent structure of RSs, and *q*-ROPFS is an improved classification approach that has attracted researchers to solve confusing and incomplete data. According to the findings, AoPS plays an important role in decision-making by aggregating data from several sources into a single value. The emergence of AoPS with *q*-ROFS hybridization with a rough set is not integrated in the *q*-ROPF context according to the best known knowledge to date. As a result, the current *q*-ROF rough research is inspired, and we will define aggregation operators depending on rough data, such as *q*-ROFRWA, *q*-ROFROWA, *q*-ROFRHWA, *q*-ROFRWG, *q*-ROFROWG, and *q*-ROFRHWG operators, under the triangular norms.

The following are the contributions to this article:

- To construct a new notion of *q*-ROPFRSs and investigate their basic operational laws
- To develop a list of aggregation operators based on algebraic and Einstein norms and also discuss related properties in detail
- To establish the entropy and distance measures to determine the unknown weight of decision makers as well as attributes' weight information
- To develop decision-making using proposed AoPS to aggregate the uncertainty in emergency decision-making real-world problems
- A numerical case study of the real-life decision-making problem concerning to agriculture farming is considered to validate the developed methodology

This article is split up as follows: basic definitions related to *q*-ROPFSs and RSs are reviewed in Section 2.  Section 3 explores the concept of the *q*-ROFRS and its basic operations.  Section 4 defines the averaging/geometric AoPS for *q*-ROPFR data. In Section 5, the entropy measure is established, and Section 6 presents the decision-making approach. Section 6 also uses the example of farming among several kinds of the agrifarming problem to explain the algorithm given in the previous section and shows that the algorithm is reasonable and applicable.  Section 7 concludes this paper.

## 2. Preliminaries

We sort out the fundamental understanding regarding the Pythagorean FS, *q*-ROPFS, and rough set in this section.

**Definition 1 (see [27]).**

Suppose a nonempty set *M*. A Pythagorean FS *Z* in the universe *M* is the following:

(1) $$\begin{array}{c} Z=\left\{\left(\delta ,\mu_{z}\left(\delta \right),\nu_{z}\left(\delta \right)\right):\delta \in M\right\}, \end{array}$$

where the values *μ*_*z*_(*δ*) ∈ [0,1] and *ν*_*z*_(*δ*) ∈ [0,1] are known as positive and negative membership grades of *δ* and (*μ*_*z*_(*δ*))^2^+(*ν*_*z*_(*δ*))^2^ ≤ 1, ∀ *δ* ∈ *M*.

**Definition 2 (see [28]).**

Let *M* be a nonempty set. A *q*-ROFS *Z* in the universe *M* is a set having the form

(2) $$\begin{array}{c} Z=\left\{\left(\delta ,\mu_{z}\left(\delta \right),\nu_{z}\left(\delta \right)\right):\delta \in M\right\}, \end{array}$$

where the values *μ*_*z*_(*δ*) ∈ [0,1] and *ν*_*z*_(*δ*) ∈ [0,1] represent positive and negative membership grades of *δ* and (*μ*_*z*_(*δ*))^*q*^+(*ν*_*z*_(*δ*))^*q*^ ≤ 1 with *q* > 2, ∀ *δ* ∈ *M*.

For simplicity, *Z*=〈*δ*, *μ*_*z*_(*δ*), *ν*_*z*_(*δ*)〉 is represented as *Z*=(*μ*_*z*_, *ν*_*z*_) and is called *q*-rung orthopair number (*q*-ROFN).

**Definition 3 .**

Suppose a universal set *M* and *ζ* ∈ *M* × *M* is a crisp relation. Then,

1. *ζ* is reflexive if (*℘*, *℘*)  ∈ *ζ*, ∀ *℘* ∈ *M*
2. *ζ* is symmetric if *℘*, ∂∈*M* and (*℘*, ∂)  ∈ *ζ*, then (∂, *℘*)  ∈ *ζ*
3. *ζ* is transitive if *℘*, ∂, *d* ∈ *M*, (*℘*, ∂)  ∈ *ζ*, and (∂, *d*) ∈ *ζ*, then (*℘*, *d*)  ∈ *ζ*

**Definition 4 .**

Suppose a nonempty set *M* and any arbitrary relation over a set *M* is *ζ* ∈ *M* × *M*. Now, define *ζ*^*∗*^ : *M*⟶*P*(*M*) as a mapping:

(3) $$\begin{array}{c} \zeta^{*}\left(℘\right)=\left\{\partial \in M:\left(℘,\partial \right)\in \zeta \right\},\text{ for }℘\in M, \end{array}$$

where *ζ*^*∗*^(*℘*) is an object's successor neighborhood *℘* w.r.t *ζ*. Crisp approximation space (AS) is defined as the pair (*M*, *ζ*). The lower and upper approximation (Lo and Up A) of £ w.r.t AS (*M*, *ζ*) for each £⊆*M* are now designated and defined as

(4) $$\begin{array}{c} \underline{\zeta }\left(L\right)=\left\{℘\in M:\zeta^{*}\left(℘\right)\subseteq L\right\},\\ \bar{\zeta }\left(L\right)=\left\{℘\in M:\zeta^{*}\left(℘\right)\cap L\neq \phi \right\}. \end{array}$$

As a result, $\left(\underline{\zeta }\left(ℒ\right),\bar{\zeta }\left(ℒ\right)\right)$ is referred to as a rough set (RS), and $\underline{\zeta }\left(ℒ\right),\bar{\zeta }\left(ℒ\right):P\left(M\right)⟶P\left(M\right)$ are upper and lower approximation operators, respectively.

**Definition 5 .**

Consider *M* to be a universe set and *ζ* ∈ *q* − *ROFS*(*M* × *M*) to be any *q*-ROF relation on a set *M*. Then,

1. *ζ* is reflexive if *μ*_*ζ*_(*℘*, *℘*)=1 and *ν*_*ζ*_(*℘*, *℘*)=0, ∀ *℘* ∈ *M*
2. *ζ* is symmetric if (*℘*, ∂) ∈ *M* × *M*, *μ*_*ζ*_(*℘*, ∂) = *μ*_*ζ*_(∂, *℘*), and *ν*_*ζ*_(*℘*, ∂) = *ν*_*ζ*_(∂, *℘*)
3. *ζ* is transitive if (*℘*, *d*) ∈ *M* × *M*, *μ*_*ζ*_(*℘*, *d*) ≥ ∨_∂∈*M*_[*μ*_*ζ*_(*℘*, ∂)∨*μ*_*ζ*_(∂, *d*)], and *ν*_*ζ*_(*℘*, *d*)=∧_∂∈*M*_[*ν*_*ζ*_(*℘*, ∂)∧*ν*_*ζ*_(∂, *d*)]

## 3. *q*−Rung Orthopair Fuzzy Rough Set

The hybrid notion of the rough set and *q*-ROFS will be developed here to acquire the notion of the *q*-ROF rough set (*q*-ROFRS) and describe its fundamental operational laws.

**Definition 6 (see [37]).**

Consider *M* to be a universe set and for any subset *ζ* ∈ *q* − ROFS(*M* × *M*) to be any nonempty *q*-ROF relation on a set *M*. The pair (*M*, *ζ*) is thus referred to as *q*-ROF AS. The lower and upper approximation (Lo and Up A) of *ℒ* w.r.t AS (*M*, *ζ*) are two *q*-ROFSs for any *ℒ*⊆*q* − ROFS(*M*), which are defined as

(5) $$\begin{array}{c} \underline{\zeta }\left(L\right)=\left\{\left(℘,\mu_{\underline{\zeta }\left(L\right)}\left(℘\right),\nu_{\underline{\zeta }\left(L\right)}\left(℘\right)\right):℘\in M\right\},\\ \bar{\zeta }\left(L\right)=\left\{\left(℘,\mu_{\bar{\zeta }\left(L\right)}\left(℘\right),\nu_{\bar{\zeta }\left(L\right)}\left(℘\right)\right):℘\in M\right\}, \end{array}$$

where

(6) $$\begin{array}{c} \mu_{\underline{\zeta }\left(L\right)}\left(℘\right)=\underset{\partial \in M}{\wedge }\left[\mu_{\zeta }\left(℘,\partial \right)\wedge \mu_{L}\left(\partial \right)\right],\\ \nu_{\underline{\zeta }\left(L\right)}\left(℘\right)=\underset{\partial \in M}{\vee }\left[\mu_{\zeta }\left(℘,\partial \right)\vee \mu_{L}\left(\partial \right)\right], \end{array}$$

(7) $$\begin{array}{c} \mu_{\bar{\zeta }\left(L\right)}\left(℘\right)=\underset{\partial \in M}{\vee }\left[\mu_{\zeta }\left(℘,\partial \right)\vee \mu_{L}\left(\partial \right)\right],\\ \nu_{\bar{\zeta }\left(L\right)}\left(℘\right)=\underset{\partial \in M}{\wedge }\left[\mu_{\zeta }\left(℘,\partial \right)\wedge \mu_{L}\left(\partial \right)\right], \end{array}$$

such that $0\leq {\left(\mu_{\underline{\zeta }\left(ℒ\right)}\left(℘\right)\right)}^{q}+{\left(\nu_{\underline{\zeta }\left(ℒ\right)}\left(℘\right)\right)}^{q}\leq 1$ and $0\leq {\left(\mu_{\bar{\zeta }\left(ℒ\right)}\left(℘\right)\right)}^{q}+{\left(\nu_{\bar{\zeta }\left(ℒ\right)}\left(℘\right)\right)}^{q}\leq 1$, *q* > 2. As $\underline{\zeta }\left(ℒ\right)$ and $\bar{\zeta }\left(ℒ\right)$ are *q*-ROFSs, $\underline{\zeta }\left(ℒ\right),\bar{\zeta }\left(ℒ\right):q-\text{ROFS}\left(M\right)⟶q-\text{ROFS}\left(M\right)$ are upper and lower approximation operators. Then, the pair $\zeta \left(ℒ\right)=\left(\underline{\zeta }\left(ℒ\right),\bar{\zeta }\left(ℒ\right)\right)=\left\{\langle ℘,\left(\mu_{\underline{\zeta }\left(ℒ\right)}\left(℘\right),\nu_{\underline{\zeta }\left(ℒ\right)}\left(℘\right)\right),\left(\mu_{\bar{\zeta }\left(ℒ\right)}\left(℘\right),\nu_{\bar{\zeta }\left(ℒ\right)}\left(℘\right)\right)\rangle :℘\in M\right\}$ is called the *q*-ROFRS.

For simplicity, $\zeta \left(ℒ\right)=\left\{\langle ℘,\left(\mu_{\underline{\zeta }\left(ℒ\right)}\left(℘\right),\nu_{\underline{\zeta }\left(ℒ\right)}\left(℘\right)\right),\left(\mu_{\bar{\zeta }\left(ℒ\right)}\left(℘\right),\nu_{\bar{\zeta }\left(ℒ\right)}\left(℘\right)\right)\rangle :℘\in M\right\}$ is denoted as $\zeta \left(ℒ\right)=\left(\left(\underline{\mu },\underline{\nu }\right),\left(\bar{\mu },\bar{\nu }\right)\right)$ known as the *q*-ROF rough value (*q* − ROFRV), and its collection is known as *q* − ROFRS(*M*).

We now set an example for better clarifying the *q*-ROFRS concept.

**Example 1 .**

Let *M*={*℘*_1_, *℘*_2_, *℘*_3_, *℘*_4_} and (*M*, *ζ*) be the *q*-ROF AS with *ζ* ∈ *q* − ROFS(*M* × *M*) being any nonempty *q*-ROF relation on a set *M* (listed in Table 1).

Now, an expert gave the optimum normal decision object *ℒ* which is a *q*-ROFS, that is,

(8) $$\begin{array}{c} L=\left\{\langle {℘}_{1},\left(\text{0}.88,\text{0}.13\right)\rangle ,\langle {℘}_{2},\left(\text{0}.57,\text{0}.36\right)\rangle ,\langle {℘}_{3},\left(\text{0}.71,\text{0}.25\right)\rangle ,\langle {℘}_{4},\left(\text{0}.84,\text{0}.15\right)\rangle \right\}. \end{array}$$

Now, to find $\underline{\zeta }\left(ℒ\right)$ and $\bar{\zeta }\left(ℒ\right)$,

(9) $$\begin{array}{c} \mu_{\underline{\zeta }\left(L\right)}\left({℘}_{1}\right)=\underset{\partial \in M}{\wedge }\left[\mu_{\zeta }\left({℘}_{1},{℘}_{1}\right)\wedge \mu_{L}\left({℘}_{1}\right)\right]\\ =\left(0.93\wedge 0.88\right)\wedge \left(0.72\wedge 0.57\right)\wedge \left(0.76\wedge 0.71\right)\wedge \left(0.57\wedge 0.84\right)\\ =0.57,\\ \nu_{\underline{\zeta }\left(L\right)}\left({℘}_{1}\right)=\underset{\partial \in M}{\vee }\left[\mu_{\zeta }\left({℘}_{1},{℘}_{1}\right)\vee \mu_{L}\left({℘}_{1}\right)\right]\\ =\left(0.11\vee 0.13\right)\vee \left(0.14\vee 0.36\right)\vee \left(0.34\vee 0.25\right)\vee \left(0.06\vee 0.15\right)\\ =0.36, \end{array}$$

(10) $$\begin{array}{c} \mu_{\bar{\zeta }\left(L\right)}\left({℘}_{1}\right)=\underset{\partial \in M}{\vee }\left[\mu_{\zeta }\left({℘}_{1},{℘}_{1}\right)\vee \mu_{L}\left({℘}_{1}\right)\right]\\ =\left(0.93\vee 0.88\right)\vee \left(0.72\vee 0.57\right)\vee \left(0.76\vee 0.71\right)\vee \left(0.57\vee 0.84\right)\\ =0.93,\\ \nu_{\bar{\zeta }\left(L\right)}\left({℘}_{1}\right)=\underset{\partial \in M}{\wedge }\left[\mu_{\zeta }\left({℘}_{1},{℘}_{1}\right)\wedge \mu_{L}\left({℘}_{1}\right)\right]\\ =\left(0.11\wedge 0.13\right)\wedge \left(0.14\wedge 0.36\right)\wedge \left(0.34\wedge 0.25\right)\wedge \left(0.06\wedge 0.15\right)\\ =0.06. \end{array}$$

Similarly, for other values,

(11) $$\begin{array}{c} \mu_{\underline{\zeta }\left(L\right)}\left({℘}_{2}\right)=0.47,\\ \nu_{\underline{\zeta }\left(L\right)}\left({℘}_{2}\right)=0.43,\\ \mu_{\underline{\zeta }\left(L\right)}\left({℘}_{3}\right)=0.57,\\ \nu_{\underline{\zeta }\left(L\right)}\left({℘}_{3}\right)=0.66,\\ \mu_{\underline{\zeta }\left(L\right)}\left({℘}_{4}\right)=0.46,\\ \nu_{\underline{\zeta }\left(L\right)}\left({℘}_{4}\right)=0.36, \end{array}$$

(12) $$\begin{array}{c} \mu_{\bar{\zeta }\left(L\right)}\left({℘}_{2}\right)=0.88,\\ \nu_{\bar{\zeta }\left(L\right)}\left({℘}_{2}\right)=0.13,\\ \mu_{\bar{\zeta }\left(L\right)}\left({℘}_{3}\right)=0.91,\\ \nu_{\bar{\zeta }\left(L\right)}\left({℘}_{3}\right)=0.06,\\ \mu_{\bar{\zeta }\left(L\right)}\left({℘}_{4}\right)=0.88,\\ \nu_{\bar{\zeta }\left(L\right)}\left({℘}_{4}\right)=0.08. \end{array}$$

Thus, the lower and upper (Lo and Up) *q*-ROFR approximation are

(13) $$\begin{array}{c} \underline{\zeta }\left(L\right)=\left\{\langle ℘,\mu_{\underline{\zeta }\left(L\right)}\left(℘\right),\nu_{\underline{\zeta }\left(L\right)}\left(℘\right)\rangle \right\}\\ =\left\{\langle {℘}_{1},0.57,0.36\rangle ,\langle {℘}_{2},0.47,0.43\rangle ,\langle {℘}_{3},0.57,0.66\rangle ,\langle {℘}_{4},0.46,0.36\rangle \right\},\\ \bar{\zeta }\left(L\right)=\left\{\langle ℘,\mu_{\bar{\zeta }\left(L\right)}\left(℘\right),\nu_{\bar{\zeta }\left(L\right)}\left(℘\right)\rangle \right\}\\ =\left\{\langle {℘}_{1},0.93,0.06\rangle ,\langle {℘}_{2},0.88,0.13\rangle ,\langle {℘}_{3},0.91,0.06\rangle ,\langle {℘}_{4},0.88,0.08\rangle \right\}. \end{array}$$

Therefore,

(14) $$\begin{array}{c} \zeta \left(L\right)=\left\{\langle ℘,\left(\mu_{\underline{\zeta }\left(L\right)}\left(℘\right),\nu_{\underline{\zeta }\left(L\right)}\left(℘\right)\right),\left(\mu_{\bar{\zeta }\left(L\right)}\left(℘\right),\nu_{\bar{\zeta }\left(L\right)}\left(℘\right)\right)\rangle :℘\in M\right\}\\ =\left\{\begin{array}{c} \langle {℘}_{1},\left(0.57,0.36\right),\left(0.93,0.06\right)\rangle ,\langle {℘}_{2},\left(0.47,0.43\right),\left(0.88,0.13\right)\rangle ,\\ \langle {℘}_{3},\left(0.57,0.66\right),\left(0.91,0.06\right)\rangle ,\langle {℘}_{4},\left(0.46,0.36\right),\left(0.88,0.08\right)\rangle \end{array}\right\}, \end{array}$$

called *q* − ROFRS.

**Definition 7 .**

Suppose $\zeta \left({ℒ}_{\text{e}}\right)=\left(\underline{\zeta }\left({ℒ}_{\text{e}}\right),\bar{\zeta }\left({ℒ}_{\text{e}}\right)\right)\;\in \;q-\text{ROFRS}\left(M\right)\;\left(e\in \mathbb{N}\right)$. The basic operational laws can be defined as follows:

1. $\zeta \left({ℒ}_{1}\right)\subseteq \zeta \left({ℒ}_{2}\right)=\left\{\left(\underline{\zeta }\left({ℒ}_{1}\right)\subseteq \underline{\zeta }\left({ℒ}_{2}\right)\right),\left(\bar{\zeta }\left({ℒ}_{1}\right)\subseteq \bar{\zeta }\left({ℒ}_{2}\right)\right)\right\}$
2. $\zeta \left({ℒ}_{1}\right)=\zeta \left({ℒ}_{2}\right)=\left\{\left(\underline{\zeta }\left({ℒ}_{1}\right)=\underline{\zeta }\left({ℒ}_{2}\right)\right),\left(\bar{\zeta }\left({ℒ}_{1}\right)=\bar{\zeta }\left({ℒ}_{2}\right)\right)\right\}$
3. $\zeta \left({ℒ}_{1}\right)\cup \zeta \left({ℒ}_{2}\right)=\left\{\left(\underline{\zeta }\left({ℒ}_{1}\right)\cup \underline{\zeta }\left({ℒ}_{2}\right)\right),\left(\bar{\zeta }\left({ℒ}_{1}\right)\cup \bar{\zeta }\left({ℒ}_{2}\right)\right)\right\}$
4. $\zeta \left({ℒ}_{1}\right)\cap \zeta \left({ℒ}_{2}\right)=\left\{\left(\underline{\zeta }\left({ℒ}_{1}\right)\cap \underline{\zeta }\left({ℒ}_{2}\right)\right),\left(\bar{\zeta }\left({ℒ}_{1}\right)\cap \bar{\zeta }\left({ℒ}_{2}\right)\right)\right\}$
5. $\zeta {\left({ℒ}_{1}\right)}^{c}=\left(\underline{\zeta }{\left({ℒ}_{\text{e}}\right)}^{c},\bar{\zeta }{\left({ℒ}_{\text{e}}\right)}^{c}\right)=\left(\left(\underline{\nu },\underline{\mu }\right),\left(\bar{\nu },\bar{\mu }\right)\right)$

**Definition 8 .**

Suppose $\zeta \left({ℒ}_{\text{e}}\right)=\left(\underline{\zeta }\left({ℒ}_{\text{e}}\right),\bar{\zeta }\left({ℒ}_{\text{e}}\right)\right)\in q-\text{ROFRS}\left(M\right)$(*e* ∈ *ℕ*). The operational laws can be defined as follows.

(1) (15) $$\begin{array}{c} \zeta \left(L_{1}\right)⊕\zeta \left(L_{2}\right)=\left\{\left(\underline{\zeta }\left(L_{1}\right)⊕\underline{\zeta }\left(L_{2}\right)\right),\left(\bar{\zeta }\left(L_{1}\right)⊕\bar{\zeta }\left(L_{2}\right)\right)\right\}\\ =\left\{\left(\underline{\mu_{1}},\underline{\nu_{1}}\right)⊕\left(\underline{\mu_{2}},\underline{\nu_{2}}\right),\left(\bar{\mu_{1}},\bar{\nu_{1}}\right)⊕\left(\bar{\mu_{2}},\bar{\nu_{2}}\right)\right\}\\ =\left\{\begin{array}{c} \left(\sqrt[{q}]{s^{-1}\left(s\left({\underline{\mu_{1}}}^{q}\right)+s\left({\underline{\mu_{2}}}^{q}\right)\right)},t^{-1}\left(t\left(\underline{\nu_{1}}\right)+t\left(\underline{\nu_{2}}\right)\right)\right),\\ \left(\sqrt[{q}]{s^{-1}\left(s\left({\bar{\mu_{1}}}^{q}\right)+s\left({\bar{\mu_{2}}}^{q}\right)\right)},t^{-1}\left(t\left(\bar{\nu_{1}}\right)+t\left(\bar{\nu_{2}}\right)\right)\right) \end{array}\right\}. \end{array}$$
(2)
  (16) $$\begin{array}{c} \zeta \left(L_{1}\right)⊗\zeta \left(L_{2}\right)=\left\{\left(\underline{\zeta }\left(L_{1}\right)⊗\underline{\zeta }\left(L_{2}\right)\right),\left(\bar{\zeta }\left(L_{1}\right)⊗\bar{\zeta }\left(L_{2}\right)\right)\right\}\\ =\left\{\left(\underline{\mu_{1}},\underline{\nu_{1}}\right)⊗\left(\underline{\mu_{2}},\underline{\nu_{2}}\right),\left(\bar{\mu_{1}},\bar{\nu_{1}}\right)⊗\left(\bar{\mu_{2}},\bar{\nu_{2}}\right)\right\}\\ =\left\{\begin{array}{c} \left(t^{-1}\left(t\left(\underline{\mu_{1}}\right)+t\left(\underline{\mu_{2}}\right)\right),\sqrt[{q}]{s^{-1}\left(s\left({\underline{\nu_{1}}}^{q}\right)+s\left({\underline{\nu_{2}}}^{q}\right)\right)}\right)\\ \left(t^{-1}\left(t\left(\bar{\mu_{1}}\right)+t\left(\bar{\mu_{2}}\right)\right),\sqrt[{q}]{s^{-1}\left(s\left({\bar{\nu_{1}}}^{q}\right)+s\left({\bar{\nu_{2}}}^{q}\right)\right)}\right) \end{array}\right\}. \end{array}$$
(3)
  (17) $$\begin{array}{c} \beta \cdot \zeta \left(L_{1}\right)=\left\{\left(\beta \cdot \underline{\zeta }\left(L_{1}\right),\beta \cdot \bar{\zeta }\left(L_{1}\right)\right)\right\}\\ =\left\{\left(\beta \cdot \left(\underline{\mu_{1}},\underline{\nu_{1}}\right),\beta \cdot \left(\bar{\mu_{1}},\bar{\nu_{1}}\right)\right)\right\}\\ =\left\{\begin{array}{c} \left(\sqrt[{q}]{s^{-1}\left(\beta s\left({\underline{\mu_{1}}}^{q}\right)\right)},t^{-1}\left(\beta t\left(\underline{\nu_{1}}\right)\right)\right)\\ \left(\sqrt[{q}]{s^{-1}\left(\beta s\left({\bar{\mu_{1}}}^{q}\right)\right)},t^{-1}\left(\beta t\left(\bar{\nu_{1}}\right)\right)\right) \end{array}\right\}. \end{array}$$
(4)
  (18) $$\begin{array}{c} {\left(\zeta \left(L_{1}\right)\right)}^{\beta }=\left\{\left({\left(\underline{\zeta }\left(L_{1}\right)\right)}^{\beta },{\left(\bar{\zeta }\left(L_{1}\right)\right)}^{\beta }\right)\right\}\\ =\left\{\left({\left(\underline{\mu_{1}},\underline{\nu_{1}}\right)}^{\beta },{\left(\bar{\mu_{1}},\bar{\nu_{1}}\right)}^{\beta }\right)\right\}\\ =\left\{\begin{array}{c} \left(t^{-1}\left(\beta t\left(\underline{\mu_{1}}\right)\right),\sqrt[{q}]{s^{-1}\left(\beta s\left({\underline{\nu_{1}}}^{q}\right)\right)}\right),\\ \left(t^{-1}\left(\beta t\left(\bar{\mu_{1}}\right)\right),\sqrt[{q}]{s^{-1}\left(\beta s\left({\bar{\nu_{1}}}^{q}\right)\right)}\right) \end{array}\right\}. \end{array}$$

Through assigning Einstein norm generator *t*(*e*_1_)=log((2 − *e*_1_)/*e*_1_) and *s*(*e*_1_)=log((1+*e*_1_)/(1 − *e*_1_)) to *t* and *s* operators,

(1)
  (19) $$\begin{array}{c} \zeta \left(L_{1}\right)⊕\zeta \left(L_{2}\right)=\left\{\left(\underline{\zeta }\left(L_{1}\right)⊕\underline{\zeta }\left(L_{2}\right)\right),\left(\bar{\zeta }\left(L_{1}\right)⊕\bar{\zeta }\left(L_{2}\right)\right)\right\}\\ =\left\{\begin{array}{c} \left(\frac{\sqrt[{q}]{{\underline{\mu_{1}}}^{q}+{\underline{\mu_{2}}}^{q}}}{\sqrt[{q}]{1+{\underline{\mu_{1}}}^{q}.{\underline{\mu_{2}}}^{q}}},\frac{\underline{\nu_{1}}.\underline{\nu_{2}}}{\sqrt[{q}]{1+\left(1-{\underline{\nu_{1}}}^{q}\right).\left(1-{\underline{\nu_{1}}}^{q}\right)}}\right),\\ \left(\frac{\sqrt[{q}]{{\bar{\mu_{1}}}^{q}+{\bar{\mu_{2}}}^{q}}}{\sqrt[{q}]{1+{\bar{\mu_{1}}}^{q}.{\bar{\mu_{2}}}^{q}}},\frac{\bar{\nu_{1}}.\bar{\nu_{2}}}{\sqrt[{q}]{1+\left(1-{\bar{\nu_{1}}}^{q}\right).\left(1-{\bar{\nu_{2}}}^{q}\right)}}\right) \end{array}\right\}. \end{array}$$
(2)
  (20) $$\begin{array}{c} \zeta \left(L_{1}\right)⊗\zeta \left(L_{2}\right)=\left\{\left(\underline{\zeta }\left(L_{1}\right)⊗\underline{\zeta }\left(L_{2}\right)\right),\left(\bar{\zeta }\left(L_{1}\right)⊗\bar{\zeta }\left(L_{2}\right)\right)\right\}\\ =\left\{\begin{array}{c} \left(\frac{\underline{\mu_{1}}.\underline{\mu_{2}}}{\sqrt[{q}]{1+\left(1-{\underline{\mu_{1}}}^{q}\right).\left(1-{\underline{\mu_{2}}}^{q}\right)}},\frac{\sqrt[{q}]{{\underline{\nu_{1}}}^{q}+{\underline{\nu_{2}}}^{q}}}{\sqrt[{q}]{1+{\underline{\nu_{1}}}^{q}.{\underline{\nu_{2}}}^{q}}}\right),\\ \left(\frac{\bar{\mu_{1}}.\bar{\mu_{2}}}{\sqrt[{q}]{1+\left(1-{\bar{\mu_{1}}}^{q}\right).\left(1-{\bar{\mu_{2}}}^{q}\right)}},\frac{\sqrt[{q}]{{\bar{\nu_{1}}}^{q}+{\bar{\nu_{2}}}^{q}}}{\sqrt[{q}]{1+{\bar{\nu_{1}}}^{q}.{\bar{\nu_{2}}}^{q}}}\right) \end{array}\right\}. \end{array}$$
(3)
  (21) $$\begin{array}{c} \beta \cdot \zeta \left(L_{1}\right)=\left\{\left(\beta \cdot \underline{\zeta }\left(L_{1}\right),\beta \cdot \bar{\zeta }\left(L_{1}\right)\right)\right\}\\ =\left\{\begin{array}{c} \left(\frac{\sqrt[{q}]{{\left(1+{\underline{\mu_{1}}}^{q}\right)}^{\beta }-{\left(1-{\underline{\mu_{1}}}^{q}\right)}^{\beta }}}{\sqrt[{q}]{{\left(1+{\underline{\mu_{1}}}^{q}\right)}^{\beta }+{\left(1-{\underline{\mu_{1}}}^{q}\right)}^{\beta }}},\frac{\sqrt[{q}]{2{\left({\underline{\nu_{1}}}^{q}\right)}^{\beta }}}{\sqrt[{q}]{{\left(2-{\underline{\nu_{1}}}^{q}\right)}^{\beta }+{\left({\underline{\nu_{1}}}^{q}\right)}^{\beta }}}\right),\\ \left(\frac{\sqrt[{q}]{{\left(1+{\bar{\mu_{1}}}^{q}\right)}^{\beta }-{\left(1-{\bar{\mu_{1}}}^{q}\right)}^{\beta }}}{\sqrt[{q}]{{\left(1+{\bar{\mu_{1}}}^{q}\right)}^{\beta }+{\left(1-{\bar{\mu_{1}}}^{q}\right)}^{\beta }}},\frac{\sqrt[{q}]{2{\left({\bar{\nu_{1}}}^{q}\right)}^{\beta }}}{\sqrt[{q}]{{\left(2-{\bar{\nu_{1}}}^{q}\right)}^{\beta }+{\left({\bar{\nu_{1}}}^{q}\right)}^{\beta }}}\right) \end{array}\right\}. \end{array}$$
(4)
  (22) $$\begin{array}{c} {\left(\zeta \left(L_{1}\right)\right)}^{\beta }=\left\{\left({\left(\underline{\zeta }\left(L_{1}\right)\right)}^{\beta },{\left(\bar{\zeta }\left(L_{1}\right)\right)}^{\beta }\right)\right\}\\ =\left\{\begin{array}{c} \left(\frac{\sqrt[{q}]{2{\left({\underline{\mu_{1}}}^{q}\right)}^{\beta }}}{\sqrt[{q}]{{\left(2-{\underline{\mu_{1}}}^{q}\right)}^{\beta }+{\left({\underline{\mu_{1}}}^{q}\right)}^{\beta }}},\frac{\sqrt[{q}]{{\left(1+{\underline{\nu_{1}}}^{q}\right)}^{\beta }-{\left(1-{\underline{\nu_{1}}}^{q}\right)}^{\beta }}}{\sqrt[{q}]{{\left(1+{\underline{\nu_{1}}}^{q}\right)}^{\beta }+{\left(1-{\underline{\nu_{1}}}^{q}\right)}^{\beta }}}\right),\\ \left(\frac{\sqrt[{q}]{2{\left({\bar{\mu_{1}}}^{q}\right)}^{\beta }}}{\sqrt[{q}]{{\left(2-{\bar{\mu_{1}}}^{q}\right)}^{\beta }+{\left({\bar{\mu_{1}}}^{q}\right)}^{\beta }}},\frac{\sqrt[{q}]{{\left(1+{\bar{\nu_{1}}}^{q}\right)}^{\beta }-{\left(1-{\bar{\nu_{1}}}^{q}\right)}^{\beta }}}{\sqrt[{q}]{{\left(1+{\bar{\nu_{1}}}^{q}\right)}^{\beta }+{\left(1-{\bar{\nu_{1}}}^{q}\right)}^{\beta }}}\right) \end{array}\right\}. \end{array}$$

To compare two or more *q*-ROFRVs, we use score function for their comparison.

**Definition 9 .**

Suppose $\zeta \left({ℒ}_{\text{e}}\right)=\left(\underline{\zeta }\left({ℒ}_{\text{e}}\right),\bar{\zeta }\left({ℒ}_{\text{e}}\right)\right)=\left(\left(\underline{\mu_{e}},\underline{\nu_{e}}\right),\left(\bar{\mu_{e}},\bar{\nu_{e}}\right)\right)\in q-\text{ROFRS}\left(M\right)\left(e\in \mathbb{N}\right)$. The following are the score (*So*) and accuracy (*Ao*) functions:

1. $So\left(\zeta \left({ℒ}_{\text{e}}\right)\right)=\left(\left(2+\underline{\mu_{e}}-\underline{\nu_{e}}+\bar{\mu_{e}}-\bar{\nu_{e}}\right)/4\right)$
2. $Ao\left(\zeta \left({ℒ}_{\text{e}}\right)\right)=\left(\underline{\mu_{e}}+\underline{\nu_{e}}+\bar{\mu_{e}}+\bar{\nu_{e}}/4\right)$

**Definition 10 .**

Suppose $\zeta \left({ℒ}_{\text{e}}\right)=\left(\underline{\zeta }\left({ℒ}_{\text{e}}\right),\bar{\zeta }\left({ℒ}_{\text{e}}\right)\right)=\left(\left(\underline{\mu_{e}},\underline{\nu_{e}}\right),\left(\bar{\mu_{e}},\bar{\nu_{e}}\right)\right)\;\in \;q-\text{ROFRS}\left(M\right)\;\left(e\in \mathbb{N}\right)$. Then,

1. If *So*(*ζ*(*ℒ*_1_)) > *So*(*ζ*(*ℒ*_2_)), ⇒ *ζ*(*ℒ*_1_) > *ζ*(*ℒ*_2_)
2. If *So*(*ζ*(*ℒ*_1_))=*So*(*ζ*(*ℒ*_2_)), ⇒
3. If *Ao*(*ζ*(*ℒ*_1_)) > *Ao*(*ζ*(*ℒ*_2_)), ⇒ *ζ*(*ℒ*_1_) > *ζ*(*ℒ*_2_)
4. If *Ao*(*ζ*(*ℒ*_1_))=*Ao*(*ζ*(*ℒ*_2_)), ⇒ *ζ*(*ℒ*_1_)=*ζ*(*ℒ*_2_)

**Proposition 1 .**

Let (*M*, *ζ*)∈*q*-ROF approximation space. Consider $\zeta \left({ℒ}_{\text{e}}\right)=\left(\underline{\zeta }\left({ℒ}_{\text{e}}\right),\bar{\zeta }\left({ℒ}_{\text{e}}\right)\right)\in q-\text{ROFRS}\left(M\right)\left(e\in \mathbb{N}\right)$. Then,

1. *ζ*(*ℒ*_1_) ∪ *ζ*(*ℒ*_2_)=*ζ*(*ℒ*_2_) ∪ *ζ*(*ℒ*_1_)
2. *ζ*(*ℒ*_1_)∩*ζ*(*ℒ*_2_)=*ζ*(*ℒ*_2_)∩*ζ*(*ℒ*_1_)
3. ((*ζ*(*ℒ*_1_))^*c*^)^*c*^=*ζ*(*ℒ*_1_), where (*ζ*(*ℒ*_1_))^*c*^ is the complement of *ζ*(*ℒ*_1_)
4. (*ζ*(*ℒ*_1_) ∪ *ζ*(*ℒ*_2_))^*c*^=(*ζ*(*ℒ*_1_))^*c*^∩(*ζ*(*ℒ*_2_))^*c*^
5. (*ζ*(*ℒ*_1_)∩*ζ*(*ℒ*_2_))^*c*^=(*ζ*(*ℒ*_1_))^*c*^ ∪ (*ζ*(*ℒ*_2_))^*c*^

**Proposition 2 .**

Consider (*M*, *ζ*)∈*q*-ROF approximation space. Consider $\zeta \left({ℒ}_{\text{e}}\right)=\left(\underline{\zeta }\left({ℒ}_{\text{e}}\right),\bar{\zeta }\left({ℒ}_{\text{e}}\right)\right)\in q-\text{ROFRS}\left(M\right)\left(e\in \mathbb{N}\right)$. The following results hold:

1. *ζ*(*ℒ*_1_) ⊕ *ζ*(*ℒ*_2_)=*ζ*(*ℒ*_2_) ⊕ *ζ*(*ℒ*_1_)
2. *ζ*(*ℒ*_1_) ⊗ *ζ*(*ℒ*_2_)=*ζ*(*ℒ*_2_) ⊗ *ζ*(*ℒ*_1_)
3. *β·*(*ζ*(*ℒ*_1_) ⊕ *ζ*(*ℒ*_2_))=(*β·ζ*(*ℒ*_1_) ⊕ *β·ζ*(*ℒ*_2_))
4. (*ζ*(*ℒ*_1_) ⊗ *ζ*(*ℒ*_2_))^*β*^=(*ζ*(*ℒ*_1_))^*β*^ ⊗ (*ζ*(*ℒ*_2_))^*β*^

## 4. *q*-Rung Orthopair Fuzzy Rough Aggregation Information

Aggregation information (AInf) plays a vital role in integrating data into a single format and solving decision-making problems (DMPs). Throughout this portion, we present a list of innovative aggregation information based on various standard-based operating regulations for *q*-ROFRVs.

### 4.1. *q*-Rung Orthopair Fuzzy Rough Averaging AInf

**Definition 11 .**

Consider (*M*, *ζ*)∈*q*-ROF AS. Let $\zeta \left({ℒ}_{\text{e}}\right)=\left(\underline{\zeta }\left({ℒ}_{\text{e}}\right),\bar{\zeta }\left({ℒ}_{\text{e}}\right)\right)\in q-\text{ROFRS}\left(M\right)\left(e\in \mathbb{N}\right)$. Then, weighted averaging AInf can be defined as in the following:

(23) $$\begin{array}{c} WA\left(\zeta \left(L_{1}\right),\zeta \left(L_{2}\right),\ldots ,\zeta \left(L_{\text{n}}\right)\right)=\left(\sum_{e=1}^{n}\beta_{e}\underline{\zeta }\left(L_{\text{e}}\right),\sum_{e=1}^{n}\beta_{e}\bar{\zeta }\left(L_{\text{e}}\right)\right), \end{array}$$

where weights of (*ζ*(*ℒ*_1_), *ζ*(*ℒ*_2_),…, *ζ*(*ℒ*_n_)) are (*β*_1_, *β*_2_,…*β*_*n*_)^*T*^, i.e., *β*_*e*_ ≥ 0; ∑_*e*=1_^*n*^*β*_*e*_=1.

**Theorem 1 .**

Consider (*M*, *ζ*)∈*q*-ROF approximation space. Consider $\zeta \left({ℒ}_{\text{e}}\right)=\left(\underline{\zeta }\left({ℒ}_{\text{e}}\right),\bar{\zeta }\left({ℒ}_{\text{e}}\right)\right)\in q-\text{ROFRS}\left(M\right)\left(e\in \mathbb{N}\right)$ and (*β*_1_, *β*_2_,…*β*_*n*_)^*T*^ is the weight information of (*ζ*(*ℒ*_1_), *ζ*(*ℒ*_2_),…, *ζ*(*ℒ*_n_)), i.e., *β*_*e*_ ≥ 0; ∑_*e*=1_^*n*^*β*_*e*_=1. Then, *WA* AInf is a mapping *D*^*n*^⟶*D*, i.e.,

(24) $$\begin{array}{c} WA\left(\zeta \left(L_{1}\right),\zeta \left(L_{2}\right),\ldots ,\zeta \left(L_{\text{n}}\right)\right)=\left(\sum_{e=1}^{n}\beta_{e}\underline{\zeta }\left(L_{\text{e}}\right),\sum_{e=1}^{n}\beta_{e}\bar{\zeta }\left(L_{\text{e}}\right)\right)\\ =\left\{\begin{array}{c} \left(\sqrt[{q}]{s^{-1}\left(\sum_{e=1}^{n}\beta_{e}s\left({\underline{\mu_{e}}}^{q}\right)\right)},t^{-1}\left(\sum_{e=1}^{n}\beta_{e}t\left(\underline{\nu_{e}}\right)\right)\right),\\ \left(\sqrt[{q}]{s^{-1}\left(\sum_{e=1}^{n}\beta_{e}s\left({\bar{\mu_{e}}}^{q}\right)\right)},t^{-1}\left(\sum_{e=1}^{n}\beta_{e}t\left(\bar{\nu_{e}}\right)\right)\right) \end{array}\right\}. \end{array}$$

For assigning values to *t* and *s* generators, we get Einstein operations for *q*-ROFRVs, similar to Einstein strict Archimedean norms.

(25) $$\begin{array}{c} WA\left(\zeta \left(L_{1}\right),\zeta \left(L_{2}\right),\ldots ,\zeta \left(L_{n}\right)\right)=\left(\sum_{e=1}^{n}\beta_{e}\underline{\zeta }\left(L_{e}\right),\sum_{e=1}^{n}\beta_{e}\bar{\zeta }\left(L_{e}\right)\right)\\ =\left\{\begin{array}{c} \left(\sqrt[{q}]{\frac{\prod_{e=1}^{n}{\left(1+{\underline{\mu_{e}}}^{q}\right)}^{\beta_{e}}\_\prod_{e=1}^{n}{\left(1-{\underline{\mu_{e}}}^{q}\right)}^{\beta_{e}}}{\prod_{e=1}^{n}{\left(1+{\underline{\mu_{e}}}^{q}\right)}^{\beta_{e}}+\prod_{e=1}^{n}{\left(1-{\underline{\mu_{e}}}^{q}\right)}^{\beta_{e}}}},\frac{\sqrt[{q}]{2\prod_{e=1}^{n}{\left({\underline{\nu_{e}}}^{q}\right)}^{\beta_{e}}}}{\sqrt[{q}]{\prod_{e=1}^{n}{\left(2-{\underline{\nu_{e}}}^{q}\right)}^{\beta_{e}}+\prod_{e=1}^{n}{\left({\underline{\nu_{e}}}^{q}\right)}^{\beta_{e}}}}\right),\\ \left(\sqrt[{q}]{\frac{\prod_{e=1}^{n}{\left(1+{\bar{\mu_{e}}}^{q}\right)}^{\beta_{e}}\_\prod_{e=1}^{n}{\left(1-{\bar{\mu_{e}}}^{q}\right)}^{\beta_{e}}}{\prod_{e=1}^{n}{\left(1+{\bar{\mu_{e}}}^{q}\right)}^{\beta_{e}}+\prod_{e=1}^{n}{\left(1-{\bar{\mu_{e}}}^{q}\right)}^{\beta_{e}}}},\frac{\sqrt[{q}]{2\prod_{e=1}^{n}{\left({\bar{\nu_{e}}}^{q}\right)}^{\beta_{e}}}}{\sqrt[{q}]{\prod_{e=1}^{n}{\left(2-{\bar{\nu_{e}}}^{q}\right)}^{\beta_{e}}+\prod_{e=1}^{n}{\left({\bar{\nu_{e}}}^{q}\right)}^{\beta_{e}}}}\right) \end{array}\right\}. \end{array}$$

**Proof**

By the induction method:

 (Case 1) Step 1: for *n*=2, we get
  (26) $$\begin{array}{c} \beta_{1}\cdot \zeta \left(L_{1}\right)=\left\{\begin{array}{c} \left(\frac{\sqrt[{q}]{{\left(1+{\bar{\mu_{1}}}^{q}\right)}^{\beta_{1}}-{\left(1-{\bar{\mu_{1}}}^{q}\right)}^{\beta_{1}}}}{\sqrt[{q}]{{\left(1+{\bar{\mu_{1}}}^{q}\right)}^{\beta_{1}}+{\left(1-{\bar{\mu_{1}}}^{q}\right)}^{\beta_{1}}}},\frac{\sqrt[{q}]{2{\left({\bar{\nu_{1}}}^{q}\right)}^{\beta_{1}}}}{\sqrt[{q}]{{\left(2-{\bar{\nu_{1}}}^{q}\right)}^{\beta_{1}}+{\left({\bar{\nu_{1}}}^{q}\right)}^{\beta_{1}}}}\right) \end{array}\right\}, \end{array}$$
  (27) $$\begin{array}{c} \beta_{2}\cdot \zeta \left(L_{2}\right)=\left\{\begin{array}{c} \left(\frac{\sqrt[{q}]{{\left(1+{\bar{\mu_{2}}}^{q}\right)}^{\beta_{2}}-{\left(1-{\bar{\mu_{2}}}^{q}\right)}^{\beta_{2}}}}{\sqrt[{q}]{{\left(1+{\bar{\mu_{2}}}^{q}\right)}^{\beta_{2}}+{\left(1-{\bar{\mu_{2}}}^{q}\right)}^{\beta_{2}}}},\frac{\sqrt[{q}]{2{\left({\bar{\nu_{2}}}^{q}\right)}^{\beta_{2}}}}{\sqrt[{q}]{{\left(2-{\bar{\nu_{2}}}^{q}\right)}^{\beta_{2}}+{\left({\bar{\nu_{2}}}^{q}\right)}^{\beta_{2}}}}\right) \end{array}\right\},\\ \left\{\begin{array}{c} \left(\frac{\sqrt[{q}]{{\left(1+{\bar{\mu_{2}}}^{q}\right)}^{\beta_{2}}-{\left(1-{\bar{\mu_{2}}}^{q}\right)}^{\beta_{2}}}}{\sqrt[{q}]{{\left(1+{\bar{\mu_{2}}}^{q}\right)}^{\beta_{2}}+{\left(1-{\bar{\mu_{2}}}^{q}\right)}^{\beta_{2}}}},\frac{\sqrt[{q}]{2{\left({\bar{\nu_{2}}}^{q}\right)}^{\beta_{2}}}}{\sqrt[{q}]{{\left(2-{\bar{\nu_{2}}}^{q}\right)}^{\beta_{2}}+{\left({\bar{\nu_{2}}}^{q}\right)}^{\beta_{2}}}}\right) \end{array}\right\}\\ =\left\{\begin{array}{c} \left(\sqrt[{q}]{\frac{\prod_{e=1}^{n}{\left(1+{\bar{\mu_{e}}}^{q}\right)}^{\beta_{e}}\_\prod_{e=1}^{n}{\left(1-{\bar{\mu_{e}}}^{q}\right)}^{\beta_{e}}}{\prod_{e=1}^{n}{\left(1+{\bar{\mu_{e}}}^{q}\right)}^{\beta_{e}}+\prod_{e=1}^{n}{\left(1-{\bar{\mu_{e}}}^{q}\right)}^{\beta_{e}}}},\frac{\sqrt[{q}]{2\prod_{e=1}^{n}{\left({\bar{\nu_{e}}}^{q}\right)}^{\beta_{e}}}}{\sqrt[{q}]{\prod_{e=1}^{n}{\left(2-{\bar{\nu_{e}}}^{q}\right)}^{\beta_{e}}+\prod_{e=1}^{n}{\left({\bar{\nu_{e}}}^{q}\right)}^{\beta_{e}}}}\right) \end{array}\right\}. \end{array}$$

 Step 2: consider for *n*=*δ*; the result is true.

(28) $$\begin{array}{c} WA\left(\zeta \left(L_{1}\right),\zeta \left(L_{2}\right),\ldots ,\zeta \left(L_{\delta }\right)\right)=\left\{\begin{array}{c} \left(\sqrt[{q}]{\frac{\prod_{e=1}^{n}{\left(1+{\underline{\mu_{e}}}^{q}\right)}^{\beta_{e}}\_\prod_{e=1}^{n}{\left(1-{\underline{\mu_{e}}}^{q}\right)}^{\beta_{e}}}{\prod_{e=1}^{n}{\left(1+{\underline{\mu_{e}}}^{q}\right)}^{\beta_{e}}+\prod_{e=1}^{n}{\left(1-{\underline{\mu_{e}}}^{q}\right)}^{\beta_{e}}}},\frac{\sqrt[{q}]{2\prod_{e=1}^{n}{\left({\underline{\nu_{e}}}^{q}\right)}^{\beta_{e}}}}{\sqrt[{q}]{\prod_{e=1}^{n}{\left(2-{\underline{\nu_{e}}}^{q}\right)}^{\beta_{e}}+\prod_{e=1}^{n}{\left({\underline{\nu_{e}}}^{q}\right)}^{\beta_{e}}}}\right),\\ \left(\sqrt[{q}]{\frac{\prod_{e=1}^{n}{\left(1+{\bar{\mu_{e}}}^{q}\right)}^{\beta_{e}}\_\prod_{e=1}^{n}{\left(1-{\bar{\mu_{e}}}^{q}\right)}^{\beta_{e}}}{\prod_{e=1}^{n}{\left(1+{\bar{\mu_{e}}}^{q}\right)}^{\beta_{e}}+\prod_{e=1}^{n}{\left(1-{\bar{\mu_{e}}}^{q}\right)}^{\beta_{e}}}},\frac{\sqrt[{q}]{2\prod_{e=1}^{n}{\left({\bar{\nu_{e}}}^{q}\right)}^{\beta_{e}}}}{\sqrt[{q}]{\prod_{e=1}^{n}{\left(2-{\bar{\nu_{e}}}^{q}\right)}^{\beta_{e}}+\prod_{e=1}^{n}{\left({\bar{\nu_{e}}}^{q}\right)}^{\beta_{e}}}}\right) \end{array}\right\}. \end{array}$$

 Step 3: consider for *n*=*δ*+1; the result is true.

(29) $$\begin{array}{c} WA\left(\zeta \left(L_{1}\right),\zeta \left(L_{2}\right),\ldots ,\zeta \left(L_{\delta +1}\right)\right)\\ =\left(\sum_{e=1}^{\delta }\beta_{e}\underline{ℋ}\left(L_{\text{e}}\right)⊕\beta_{\delta +1}\underline{\zeta }\left(L_{\delta +1}\right),\sum_{e=1}^{\delta }\beta_{e}\bar{\zeta }\left(L_{\text{e}}\right)⊕\beta_{\delta +1}\bar{\zeta }\left(L_{\delta +1}\right)\right)\\ =\left\{\begin{array}{c} \left(\begin{array}{c} \sqrt[{q}]{\frac{\prod_{e=1}^{\delta }{\left(1+{\underline{\mu_{e}}}^{q}\right)}^{\beta_{e}}\_\prod_{e=1}^{\delta }{\left(1-{\underline{\mu_{e}}}^{q}\right)}^{\beta_{e}}}{\prod_{e=1}^{\delta }{\left(1+{\underline{\mu_{e}}}^{q}\right)}^{\beta_{e}}+\prod_{e=1}^{\delta }{\left(1-{\underline{\mu_{e}}}^{q}\right)}^{\beta_{e}}}},\\ \frac{\sqrt[{q}]{2\prod_{e=1}^{\delta }{\left({\underline{\nu_{e}}}^{q}\right)}^{\beta_{e}}}}{\sqrt[{q}]{\prod_{e=1}^{\delta }{\left(2-{\underline{\nu_{e}}}^{q}\right)}^{\beta_{e}}+\prod_{e=1}^{\delta }{\left({\underline{\nu_{e}}}^{q}\right)}^{\beta_{e}}}} \end{array}\right)⊕\left(\begin{array}{c} \sqrt[{q}]{\frac{{\left(1+{\underline{\mu_{\delta +1}}}^{q}\right)}^{\beta_{\delta +1}}\_{\left(1-{\underline{\mu_{\delta +1}}}^{q}\right)}^{\beta_{\delta +1}}}{{\left(1+{\underline{\mu_{\delta +1}}}^{q}\right)}^{\beta_{\delta +1}}+{\left(1-{\underline{\mu_{\delta +1}}}^{q}\right)}^{\beta_{\delta +1}}}},\\ \frac{\sqrt[{q}]{2{\left({\underline{\nu_{\delta +1}}}^{q}\right)}^{\beta_{\delta +1}}}}{\sqrt[{q}]{{\left(2-{\underline{\nu_{\delta +1}}}^{q}\right)}^{\beta_{\delta +1}}+{\left({\underline{\nu_{\delta +1}}}^{q}\right)}^{\beta_{\delta +1}}}} \end{array}\right),\\ \left(\begin{array}{c} \sqrt[{q}]{\frac{\prod_{e=1}^{n}{\left(1+{\bar{\mu_{e}}}^{q}\right)}^{\beta_{e}}\_\prod_{e=1}^{n}{\left(1-{\bar{\mu_{e}}}^{q}\right)}^{\beta_{e}}}{\prod_{e=1}^{n}{\left(1+{\bar{\mu_{e}}}^{q}\right)}^{\beta_{e}}+\prod_{e=1}^{n}{\left(1-{\bar{\mu_{e}}}^{q}\right)}^{\beta_{e}}}},\\ \left.\frac{\sqrt[{q}]{2\prod_{e=1}^{n}{\left({\bar{\nu_{e}}}^{q}\right)}^{\beta_{e}}}}{\sqrt[{q}]{\prod_{e=1}^{n}{\left(2-{\bar{\nu_{e}}}^{q}\right)}^{\beta_{e}}+\prod_{e=1}^{n}{\left({\bar{\nu_{e}}}^{q}\right)}^{\beta_{e}}}}\right] \end{array}\right)⊕\left(\begin{array}{c} \sqrt[{q}]{\frac{{\left(1+{\bar{\mu_{\delta +1}}}^{q}\right)}^{\beta_{\delta +1}}\_{\left(1-{\bar{\mu_{\delta +1}}}^{q}\right)}^{\beta_{\delta +1}}}{{\left(1+{\bar{\mu_{\delta +1}}}^{q}\right)}^{\beta_{\delta +1}}+{\left(1-{\bar{\mu_{\delta +1}}}^{q}\right)}^{\beta_{\delta +1}}}},\\ \frac{\sqrt[{q}]{2{\left({\bar{\nu_{\delta +1}}}^{q}\right)}^{\beta_{\delta +1}}}}{\sqrt[{q}]{{\left(2-{\bar{\nu_{\delta +1}}}^{q}\right)}^{\beta_{\delta +1}}+{\left({\bar{\nu_{\delta +1}}}^{q}\right)}^{\beta_{\delta +1}}}} \end{array}\right) \end{array}\right\}\\ =\left\{\begin{array}{c} \left(\sqrt[{q}]{\frac{\prod_{e=1}^{\delta +1}{\left(1+{\underline{\mu_{e}}}^{q}\right)}^{\beta_{e}}\_\prod_{e=1}^{\delta +1}{\left(1-{\underline{\mu_{e}}}^{q}\right)}^{\beta_{e}}}{\prod_{e=1}^{\delta +1}{\left(1+{\underline{\mu_{e}}}^{q}\right)}^{\beta_{e}}+\prod_{e=1}^{\delta +1}{\left(1-{\underline{\mu_{e}}}^{q}\right)}^{\beta_{e}}}},\frac{\sqrt[{q}]{2\prod_{e=1}^{\delta +1}{\left({\underline{\nu_{e}}}^{q}\right)}^{\beta_{e}}}}{\sqrt[{q}]{\prod_{e=1}^{\delta +1}{\left(2-{\underline{\nu_{e}}}^{q}\right)}^{\beta_{e}}+\prod_{e=1}^{\delta +1}{\left({\underline{\nu_{e}}}^{q}\right)}^{\beta_{e}}}}\right),\\ \left(\sqrt[{q}]{\frac{\prod_{e=1}^{\delta +1}{\left(1+{\bar{\mu_{e}}}^{q}\right)}^{\beta_{e}}\_\prod_{e=1}^{\delta +1}{\left(1+{\bar{\mu_{e}}}^{q}\right)}^{\beta_{e}}}{\prod_{e=1}^{\delta +1}{\left(1+{\bar{\mu_{e}}}^{q}\right)}^{\beta_{e}}+\prod_{e=1}^{\delta +1}{\left(1+{\bar{\mu_{e}}}^{q}\right)}^{\beta_{e}}}},\frac{\sqrt[{q}]{2\prod_{e=1}^{\delta +1}{\left({\bar{\nu_{e}}}^{q}\right)}^{\beta_{e}}}}{\sqrt[{q}]{\prod_{e=1}^{\delta +1}{\left(2-{\bar{\nu_{e}}}^{q}\right)}^{\beta_{e}}+\prod_{e=1}^{\delta +1}{\left({\bar{\nu_{e}}}^{q}\right)}^{\beta_{e}}}}\right) \end{array}\right\}. \end{array}$$

Hence, ∀ positive integers, the given result is valid.

(30) $$\begin{array}{c} WA\left(\zeta \left(L_{1}\right),\zeta \left(L_{2}\right),\ldots ,\zeta \left(L_{n}\right)\right)=\left\{\begin{array}{c} \left(\sqrt[{q}]{\frac{\prod_{e=1}^{n}{\left(1+{\underline{\mu_{e}}}^{q}\right)}^{\beta_{e}}\_\prod_{e=1}^{n}{\left(1-{\underline{\mu_{e}}}^{q}\right)}^{\beta_{e}}}{\prod_{e=1}^{n}{\left(1+{\underline{\mu_{e}}}^{q}\right)}^{\beta_{e}}+\prod_{e=1}^{n}{\left(1-{\underline{\mu_{e}}}^{q}\right)}^{\beta_{e}}}},\frac{\sqrt[{q}]{2\prod_{e=1}^{n}{\left({\underline{\nu_{e}}}^{q}\right)}^{\beta_{e}}}}{\sqrt[{q}]{\prod_{e=1}^{n}{\left(2-{\underline{\nu_{e}}}^{q}\right)}^{\beta_{e}}+\prod_{e=1}^{n}{\left({\underline{\nu_{e}}}^{q}\right)}^{\beta_{e}}}}\right),\\ \left(\sqrt[{q}]{\frac{\prod_{e=1}^{n}{\left(1+{\bar{\mu_{e}}}^{q}\right)}^{\beta_{e}}\_\prod_{e=1}^{n}{\left(1-{\bar{\mu_{e}}}^{q}\right)}^{\beta_{e}}}{\prod_{e=1}^{n}{\left(1+{\bar{\mu_{e}}}^{q}\right)}^{\beta_{e}}+\prod_{e=1}^{n}{\left(1-{\bar{\mu_{e}}}^{q}\right)}^{\beta_{e}}}},\frac{\sqrt[{q}]{2\prod_{e=1}^{n}{\left({\bar{\nu_{e}}}^{q}\right)}^{\beta_{e}}}}{\sqrt[{q}]{\prod_{e=1}^{n}{\left(2-{\bar{\nu_{e}}}^{q}\right)}^{\beta_{e}}+\prod_{e=1}^{n}{\left({\bar{\nu_{e}}}^{q}\right)}^{\beta_{e}}}}\right) \end{array}\right\}, \end{array}$$

hence proved.

From the above analysis, $\zeta \left(ℒ\right)=\left(\underline{\zeta }\left(ℒ\right),\bar{\zeta }\left(ℒ\right)\right)$ is the *q*-ROFRV. So, by Definition 8, $\left(\sum_{e=1}^{n}\beta_{e}\underline{\zeta }\left({ℒ}_{\text{e}}\right),\sum_{e=1}^{n}\beta_{e}\bar{\zeta }\left({ℒ}_{\text{e}}\right)\right)$ are also *q*-ROFRVs. Therefore, *WA*(*ζ*(*ℒ*_1_), *ζ*(*ℒ*_2_),…, *ζ*(*ℒ*_n_)) is also a *q*-ROFRV under *q*-ROF AS (*M*, *ζ*).

Some important properties of the *q*-ROF rough weighted averaging operator are initiated in Theorem 2.

**Theorem 2 .**

Consider (*M*, *ζ*)∈*q*-ROF AS. Let $\zeta \left({ℒ}_{\text{e}}\right)=\left(\underline{\zeta }\left({ℒ}_{\text{e}}\right),\bar{\zeta }\left({ℒ}_{\text{e}}\right)\right)\in q-\text{ROFRS}\left(M\right)\left(e\in \mathbb{N}\right)$ and (*β*_1_, *β*_2_,…*β*_*n*_)^*T*^ be the weight information of (*ζ*(*ℒ*_1_), *ζ*(*ℒ*_2_),…, *ζ*(*ℒ*_n_)), i.e., *β*_*e*_ ≥ 0; ∑_*e*=1_^*n*^*β*_*e*_=1. Then, some important properties of the *q*-ROF rough weighted averaging operator are described as follows:

(1) Idempotency: if $\zeta \left({ℒ}_{\text{e}}\right)=\zeta \left(ℒ\right)=\left(\underline{\zeta }\left(ℒ\right),\bar{\zeta }\left(ℒ\right)\right)$∀ *e* ∈ *ℕ*, then
  (31) $$\begin{array}{c} WA\left(\zeta \left(L_{1}\right),\zeta \left(L_{2}\right),\ldots ,\zeta \left(L_{\text{n}}\right)\right)=\zeta \left(L\right). \end{array}$$
(2) Boundedness: let ${\left(\zeta \left(ℒ\right)\right)}^{-}=\left(\underset{e}{\min}\underline{\zeta }\left({ℒ}_{\text{e}}\right),\underset{e}{\max}\bar{\zeta }\left({ℒ}_{\text{e}}\right)\right)$ and ${\left(\zeta \left(ℒ\right)\right)}^{+}=\left(\underset{e}{\max}\underline{\zeta }\left({ℒ}_{\text{e}}\right),\underset{e}{\min}\bar{\zeta }\left({ℒ}_{\text{e}}\right)\right)$. Then,
  (32) $$\begin{array}{c} {\left(\zeta \left(L\right)\right)}^{-}\leq WA\left(\zeta \left(L_{1}\right),\zeta \left(L_{2}\right),\ldots ,\zeta \left(L_{\text{n}}\right)\right)\leq {\left(\zeta \left(L\right)\right)}^{+}. \end{array}$$
(3) Monotonicity: let $P\left({ℒ}_{\text{e}}\right)=\left(\underline{P}\left({ℒ}_{\text{e}}\right),\bar{P}\left({ℒ}_{\text{e}}\right)\right)\in q-\text{ROFRS}\left(M\right)\left(e\in \mathbb{N}\right)$ such that $\underline{P}\left({ℒ}_{\text{e}}\right)\leq \underline{\zeta }\left({ℒ}_{\text{e}}\right)$ and $\bar{P}\left({ℒ}_{\text{e}}\right)\leq \bar{\zeta }\left({ℒ}_{\text{e}}\right)$. Then,
  (33) $$\begin{array}{c} WA\left(P\left(L_{1}\right),P\left(L_{2}\right),\ldots ,P\left(L_{\text{n}}\right)\right)\leq WA\left(\zeta \left(L_{1}\right),\zeta \left(L_{2}\right),\ldots ,\zeta \left(L_{\text{n}}\right)\right). \end{array}$$

**Proof**

Straightforward.

**Definition 12 .**

Consider (*M*, *ζ*)∈*q*-ROF AS. Let $\zeta \left({ℒ}_{\text{e}}\right)=\left(\underline{\zeta }\left({ℒ}_{\text{e}}\right),\bar{\zeta }\left({ℒ}_{\text{e}}\right)\right)\in q-\text{ROFRS}\left(M\right)\left(e\in \mathbb{N}\right)$. Then, ordered weighted averaging AInf can be defined as in the following:

(34) $$\begin{array}{c} OWA\left(\zeta \left(L_{1}\right),\zeta \left(L_{2}\right),\ldots ,\zeta \left(L_{\text{n}}\right)\right)=\left(\sum_{e=1}^{n}\beta_{e}\underline{\zeta }\left(L_{\xi \left(\text{e}\right)}\right),\sum_{e=1}^{n}\beta_{e}\bar{\zeta }\left(L_{\xi \left(\text{e}\right)}\right)\right), \end{array}$$

where according to (*ξ*(1), *ξ*(2), *ξ*(3),…, *ξ*(*n*)), *ξ*(*e*) is represented as the order, and the weight of (*ζ*(*ℒ*_1_), *ζ*(*ℒ*_2_),…, *ζ*(*ℒ*_n_)) is (*β*_1_, *β*_2_,…*β*_*n*_)^*T*^, i.e., *β*_*e*_ ≥ 0; ∑_*e*=1_^*n*^*β*_*e*_=1.

**Theorem 3 .**

Consider (*M*, *ζ*)∈*q*-ROF AS. Let $\zeta \left({ℒ}_{\text{e}}\right)=\left(\underline{\zeta }\left({ℒ}_{\text{e}}\right),\bar{\zeta }\left({ℒ}_{\text{e}}\right)\right)\in q-\text{ROFRS}\left(M\right)\left(e\in \mathbb{N}\right)$ and the weight of (*ζ*(*ℒ*_1_), *ζ*(*ℒ*_2_),…, *ζ*(*ℒ*_n_)) be (*β*_1_, *β*_2_,…*β*_*n*_)^*T*^, i.e., *β*_*e*_ ≥ 0; ∑_*e*=1_^*n*^*β*_*e*_=1. Then, *OWA* AInf is a transformation *D*^*n*^⟶*D*, i.e.,

(35) $$\begin{array}{c} OWA\left(\zeta \left(L_{1}\right),\zeta \left(L_{2}\right),\ldots ,\zeta \left(L_{\text{n}}\right)\right)=\left(\sum_{e=1}^{n}\beta_{e}\underline{\zeta }\left(L_{\xi \left(\text{e}\right)}\right),\sum_{e=1}^{n}\beta_{e}\bar{\zeta }\left(L_{\xi \left(\text{e}\right)}\right)\right)\\ =\left\{\begin{array}{c} \left(\sqrt[{q}]{s^{-1}\left(\sum_{e=1}^{n}\beta_{e}s\left({\underline{\mu_{\xi \left(e\right)}}}^{q}\right)\right)},t^{-1}\left(\sum_{e=1}^{n}\beta_{e}t\left(\underline{\nu_{\xi \left(e\right)}}\right)\right)\right),\\ \left(\sqrt[{q}]{s^{-1}\left(\sum_{e=1}^{n}\beta_{e}s\left({\bar{\mu_{\xi \left(e\right)}}}^{q}\right)\right)},t^{-1}\left(\sum_{e=1}^{n}\beta_{e}t\left(\bar{\nu_{\xi \left(e\right)}}\right)\right)\right) \end{array}\right\}. \end{array}$$

For assigning values to *t* and *s* generators, we get Einstein operations for *q*-ROFRVs, similar to Einstein strict Archimedean norms.

(36) $$\begin{array}{c} OWA\left(\zeta \left(L_{1}\right),\zeta \left(L_{2}\right),...,\zeta \left(L_{n}\right)\right)=\left(\sum_{e=1}^{n}\beta_{e}\underline{\zeta }\left(L_{\xi \left(e\right)}\right),\sum_{e=1}^{n}\beta_{e}\bar{\zeta }\left(L_{\xi \left(e\right)}\right)\right)\\ =\left\{\begin{array}{c} \left(\sqrt[{q}]{\frac{\prod_{e=1}^{n}{\left(1+{\underline{\mu_{\xi \left(e\right)}}}^{q}\right)}^{\beta_{e}}\_\prod_{e=1}^{n}{\left(1-{\underline{\mu_{\xi \left(e\right)}}}^{q}\right)}^{\beta_{e}}}{\prod_{e=1}^{n}{\left(1+{\underline{\mu_{\xi \left(e\right)}}}^{q}\right)}^{\beta_{e}}+\overset{n}{\underset{e=1}{\prod }}\prod_{e=1}^{n}{\left(1-{\underline{\mu_{\xi \left(e\right)}}}^{q}\right)}^{\beta_{e}}}},\frac{\sqrt[{q}]{2\prod_{e=1}^{n}{\left({\left(\underline{\nu_{\xi \left(e\right)}}\right)}^{q}\right)}^{\beta_{e}}}}{\sqrt[{q}]{\prod_{e=1}^{n}{\left(2-{\underline{\nu_{\xi \left(e\right)}}}^{q}\right)}^{\beta_{e}}+\prod_{e=1}^{n}{\left({\left(\underline{\nu_{\xi \left(e\right)}}\right)}^{q}\right)}^{\beta_{e}}}}\right),\\ \left(\sqrt[{q}]{\frac{\prod_{e=1}^{n}{\left(1+{\bar{\mu_{\xi \left(e\right)}}}^{q}\right)}^{\beta_{e}}\_\prod_{e=1}^{n}{\left(1-{\bar{\mu_{\xi \left(e\right)}}}^{q}\right)}^{\beta_{e}}}{\prod_{e=1}^{n}{\left(1+{\bar{\mu_{\xi \left(e\right)}}}^{q}\right)}^{\beta_{e}}+\prod_{e=1}^{n}{\left(1-{\bar{\mu_{\xi \left(e\right)}}}^{q}\right)}^{\beta_{e}}}},\frac{\sqrt[{q}]{2\prod_{e=1}^{n}{\left({\left(\bar{\nu_{\xi \left(e\right)}}\right)}^{q}\right)}^{\beta_{e}}}}{\sqrt[{q}]{\prod_{e=1}^{n}{\left(2-{\bar{\nu_{\xi \left(e\right)}}}^{q}\right)}^{\beta_{e}}+\prod_{e=1}^{n}{\left({\left(\bar{\nu_{\xi \left(e\right)}}\right)}^{q}\right)}^{\beta_{e}}}}\right) \end{array}\right\}. \end{array}$$

**Proof**

Follow from Theorem 1.

**Theorem 4 .**

Consider (*M*, *ζ*) to be a *q*-ROF AS. Consider $\zeta \left({ℒ}_{\text{e}}\right)=\left(\underline{\zeta }\left({ℒ}_{\text{e}}\right),\bar{\zeta }\left({ℒ}_{\text{e}}\right)\right)\;\in \;q-\text{ROFRS}\left(M\right)\;\left(e\in \mathbb{N}\right)$ and the weight of (*ζ*(*ℒ*_1_), *ζ*(*ℒ*_2_),…, *ζ*(*ℒ*_n_)) be (*β*_1_, *β*_2_,…*β*_*n*_)^*T*^, i.e., *β*_*e*_ ≥ 0; ∑_*e*=1_^*n*^*β*_*e*_=1. Then, some important properties of the *q*-ROF rough ordered weighted averaging operator are described as follows:

(1) Idempotency: if $\zeta \left({ℒ}_{\text{e}}\right)=\zeta \left(ℒ\right)=\left(\underline{\zeta }\left(ℒ\right),\bar{\zeta }\left(ℒ\right)\right)$∀ *e* ∈ *ℕ*, then
  (37) $$\begin{array}{c} OWA\left(\zeta \left(L_{1}\right),\zeta \left(L_{2}\right),\ldots ,\zeta \left(L_{\text{n}}\right)\right)=\zeta \left(L\right). \end{array}$$
(2) Boundedness: let ${\left(\zeta \left(ℒ\right)\right)}^{-}=\left(\underset{e}{\min}\underline{\zeta }\left({ℒ}_{\text{e}}\right),\underset{e}{\max}\bar{\zeta }\left({ℒ}_{\text{e}}\right)\right)$ and ${\left(\zeta \left(ℒ\right)\right)}^{+}=\left(\underset{e}{\max}\underline{\zeta }\left({ℒ}_{\text{e}}\right),\underset{e}{\min}\bar{\zeta }\left({ℒ}_{\text{e}}\right)\right)$. Then,
  (38) $$\begin{array}{c} {\left(\zeta \left(L\right)\right)}^{-}\leq OWA\left(\zeta \left(L_{1}\right),\zeta \left(L_{2}\right),\ldots ,\zeta \left(L_{\text{n}}\right)\right)\leq {\left(\zeta \left(L\right)\right)}^{+}. \end{array}$$
(3) Monotonicity: let $P\left({ℒ}_{\text{e}}\right)=\left(\underline{P}\left({ℒ}_{\text{e}}\right),\bar{P}\left({ℒ}_{\text{e}}\right)\right)\in q-\text{ROFRS}\left(M\right)\left(e\in \mathbb{N}\right)$ such that $\underline{P}\left({ℒ}_{\text{e}}\right)\leq \underline{\zeta }\left({ℒ}_{\text{e}}\right)$ and $\bar{P}\left({ℒ}_{\text{e}}\right)\leq \bar{\zeta }\left({ℒ}_{\text{e}}\right)$. Then,
  (39) $$\begin{array}{c} OWA\left(P\left(L_{1}\right),P\left(L_{2}\right),\ldots ,P\left(L_{\text{n}}\right)\right)\leq OWA\left(\zeta \left(L_{1}\right),\zeta \left(L_{2}\right),\ldots ,\zeta \left(L_{\text{n}}\right)\right). \end{array}$$

**Proof**

Follow from Theorem 2.

**Definition 13 .**

Consider (*M*, *ζ*)∈*q*-ROF AS. Consider $\zeta \left({ℒ}_{\text{e}}\right)=\left(\underline{\zeta }\left({ℒ}_{\text{e}}\right),\bar{\zeta }\left({ℒ}_{\text{e}}\right)\right)\in q-\text{ROFRS}\left(M\right)\left(e\in \mathbb{N}\right)$. Then, hybrid weighted averaging (HWA) AInf is defined as in the following:

(40) $$\begin{array}{c} HWA\left(\zeta \left(L_{1}\right),\zeta \left(L_{2}\right),\ldots ,\zeta \left(L_{\text{n}}\right)\right)=\left(\sum_{e=1}^{n}\eta_{e}\underline{\zeta }\left(L_{\xi \left(\text{e}\right)}^{\prime }\right),\sum_{e=1}^{n}\eta_{e}\bar{\zeta }\left(L_{\xi \left(\text{e}\right)}^{\prime }\right)\right), \end{array}$$

where the order according to (*ξ*(1), *ξ*(2), *ξ*(3),…, *ξ*(*n*)) is represented by *ξ*(*e*) such that $\underline{\zeta }\left({ℒ}_{\xi \left(\text{e}\right)}^{\prime }\right)\left(\underline{\zeta }\left({ℒ}_{\xi \left(\text{e}\right)}^{\prime }\right)=n\beta_{e}\underline{\zeta }\left({ℒ}_{\text{e}}\right):e\in \mathbb{N}\right)$ and $\bar{\zeta }\left({ℒ}_{\xi \left(\text{e}\right)}^{\prime }\right)\left(\bar{\zeta }\left({ℒ}_{\xi \left(\text{e}\right)}^{\prime }\right)=n\beta_{e}\bar{\zeta }\left({ℒ}_{\text{e}}\right):e\in \mathbb{N}\right)$, and the weight of (*ζ*(*ℒ*_1_), *ζ*(*ℒ*_2_),…, *ζ*(*ℒ*_n_)) is (*β*_1_, *β*_2_,…*β*_*n*_)^*T*^, i.e., *β*_*e*_ ≥ 0; ∑_*e*=1_^*n*^*β*_*e*_=1. Also, (*η*_1_, *η*_2_,…*η*_*n*_)^*T*^ represent the corresponding weight of (*ζ*(*ℒ*_1_), *ζ*(*ℒ*_2_),…, *ζ*(*ℒ*_n_)), i.e., *η*_*e*_ ≥ 0; ∑_*e*=1_^*n*^*η*_*e*_=1.

**Theorem 5 .**

Consider (*M*, *ζ*)∈*q*-ROF AS. Consider $\zeta \left({ℒ}_{\text{e}}\right)=\left(\underline{\zeta }\left({ℒ}_{\text{e}}\right),\bar{\zeta }\left({ℒ}_{\text{e}}\right)\right)\;\in \;q-\text{ROFRS}\left(M\right)\;\left(e\in \mathbb{N}\right)$ and (*β*_1_, *β*_2_,…*β*_*n*_)^*T*^ to be the weight of (*ζ*(*ℒ*_1_), *ζ*(*ℒ*_2_),…, *ζ*(*ℒ*_n_)), i.e., *β*_*e*_ ≥ 0; ∑_*e*=1_^*n*^*β*_*e*_=1. Then, *HWA* AInf is a mapping *D*^*n*^⟶*D* with associated weight (*η*_1_, *η*_2_,…*η*_*n*_)^*T*^, i.e., *η*_*e*_ ≥ 0, ∑_*e*=1_^*n*^*η*_*e*_=1, such that

(41) $$\begin{array}{c} HWA\left(\zeta \left(L_{1}\right),\zeta \left(L_{2}\right),\ldots ,\zeta \left(L_{\text{n}}\right)\right)=\left(\sum_{e=1}^{n}\eta_{e}\underline{\zeta }\left(L_{\xi \left(\text{e}\right)}^{\prime }\right),\sum_{e=1}^{n}\eta_{e}\bar{\zeta }\left(L_{\xi \left(\text{e}\right)}^{\prime }\right)\right)\\ =\left\{\begin{array}{c} \left(\sqrt[{q}]{s^{-1}\left(\sum_{e=1}^{n}\eta_{e}s\left({\underline{\mu_{\xi \left(e\right)}^{\prime }}}^{q}\right)\right)},t^{-1}\left(\sum_{e=1}^{n}\eta_{e}t\left(\underline{\nu_{\xi \left(e\right)}^{\prime }}\right)\right)\right),\\ \left(\sqrt[{q}]{s^{-1}\left(\sum_{e=1}^{n}\eta_{e}s\left({\bar{\mu_{\xi \left(e\right)}^{\prime }}}^{q}\right)\right)},t^{-1}\left(\sum_{e=1}^{n}\eta_{e}t\left(\bar{\nu_{\xi \left(e\right)}^{\prime }}\right)\right)\right) \end{array}\right\}. \end{array}$$

For assigning values to *t* and *s* generators, we get Einstein operations for *q*-ROFRVs, similar to Einstein strict Archimedean norms.

(42) $$\begin{array}{c} HWA\left(\zeta \left(L_{1}\right),\zeta \left(L_{2}\right),\ldots ,\zeta \left(L_{\text{n}}\right)\right)=\left(\sum_{e=1}^{n}\eta_{e}\underline{\zeta }\left(L_{\xi \left(\text{e}\right)}^{\prime }\right),\sum_{e=1}^{n}\eta_{e}\bar{\zeta }\left(L_{\xi \left(\text{e}\right)}^{\prime }\right)\right)\\ =\left\{\begin{array}{c} \left(\sqrt[{q}]{\frac{\prod_{e=1}^{n}{\left(1+{\underline{\mu_{\xi \left(e\right)}}}^{q}\right)}^{\eta_{e}}\_\prod_{e=1}^{n}{\left(1-{\underline{\mu_{\xi \left(e\right)}}}^{q}\right)}^{\eta_{e}}}{\prod_{e=1}^{n}{\left(1+{\underline{\mu_{\xi \left(e\right)}}}^{q}\right)}^{\eta_{e}}+\overset{n}{\underset{e=1}{\prod }}\prod_{e=1}^{n}{\left(1-{\underline{\mu_{\xi \left(e\right)}}}^{q}\right)}^{\eta_{e}}}},\frac{\sqrt[{q}]{2\prod_{e=1}^{n}{\left({\left(\underline{\nu_{\xi \left(e\right)}}\right)}^{q}\right)}^{\eta_{e}}}}{\sqrt[{q}]{\prod_{e=1}^{n}{\left(2-{\underline{\nu_{\xi \left(e\right)}}}^{q}\right)}^{\eta_{e}}+\prod_{e=1}^{n}{\left({\left(\underline{\nu_{\xi \left(e\right)}}\right)}^{q}\right)}^{\eta_{e}}}}\right),\\ \left(\sqrt[{q}]{\frac{\prod_{e=1}^{n}{\left(1+{\bar{\mu_{\xi \left(e\right)}}}^{q}\right)}^{\eta_{e}}\_\prod_{e=1}^{n}{\left(1-{\bar{\mu_{\xi \left(e\right)}}}^{q}\right)}^{\eta_{e}}}{\prod_{e=1}^{n}{\left(1+{\bar{\mu_{\xi \left(e\right)}}}^{q}\right)}^{\eta_{e}}+\prod_{e=1}^{n}{\left(1-{\bar{\mu_{\xi \left(e\right)}}}^{q}\right)}^{\eta_{e}}}},\frac{\sqrt[{q}]{2\prod_{e=1}^{n}{\left({\left(\bar{\nu_{\xi \left(e\right)}}\right)}^{q}\right)}^{\eta_{e}}}}{\sqrt[{q}]{\prod_{e=1}^{n}{\left(2-{\bar{\nu_{\xi \left(e\right)}}}^{q}\right)}^{\eta_{e}}+\prod_{e=1}^{n}{\left({\left(\bar{\nu_{\xi \left(e\right)}}\right)}^{q}\right)}^{\eta_{e}}}}\right) \end{array}\right\}. \end{array}$$

**Proof**

Follow from Theorem 1.

**Theorem 6 .**

Consider that (*M*, *ζ*)∈*q*-ROF approximation space. Let $\zeta \left({ℒ}_{\text{e}}\right)=\left(\underline{\zeta }\left({ℒ}_{\text{e}}\right),\bar{\zeta }\left({ℒ}_{\text{e}}\right)\right)\;\in \;q-\text{ROFRS}\left(M\right)\left(e\in \mathbb{N}\right)$ and weight of (*ζ*(*ℒ*_1_), *ζ*(*ℒ*_2_),…, *ζ*(*ℒ*_n_)) be (*β*_1_, *β*_2_,…*β*_*n*_)^*T*^, i.e., *β*_*e*_ ≥ 0; ∑_*e*=1_^*n*^*β*_*e*_=1. Then, some important properties of the *q*-ROF rough hybrid weighted averaging operator are described as follows:

(1) Idempotency: if $\zeta \left({ℒ}_{\text{e}}\right)=\zeta \left(ℒ\right)=\left(\underline{\zeta }\left(ℒ\right),\bar{\zeta }\left(ℒ\right)\right)$∀ *e* ∈ *ℕ*, then
  (43) $$\begin{array}{c} HWA\left(\zeta \left(L_{1}\right),\zeta \left(L_{2}\right),\ldots ,\zeta \left(L_{\text{n}}\right)\right)=\zeta \left(L\right). \end{array}$$
(2) Boundedness: let ${\left(\zeta \left(ℒ\right)\right)}^{-}=\left(\underset{e}{\min}\underline{\zeta }\left({ℒ}_{\text{e}}\right),\underset{e}{\max}\bar{\zeta }\left({ℒ}_{\text{e}}\right)\right)$ and ${\left(\zeta \left(ℒ\right)\right)}^{+}=\left(\underset{e}{\max}\underline{\zeta }\left({ℒ}_{\text{e}}\right),\underset{e}{\min}\bar{\zeta }\left({ℒ}_{\text{e}}\right)\right)$. Then,
  (44) $$\begin{array}{c} {\left(\zeta \left(L\right)\right)}^{-}\leq HWA\left(\zeta \left(L_{1}\right),\zeta \left(L_{2}\right),\ldots ,\zeta \left(L_{\text{n}}\right)\right)\leq {\left(\zeta \left(L\right)\right)}^{+}. \end{array}$$
(3) Monotonicity: let $P\left({ℒ}_{\text{e}}\right)=\left(\underline{P}\left({ℒ}_{\text{e}}\right),\bar{P}\left({ℒ}_{\text{e}}\right)\right)\in q-\text{ROFRS}\left(M\right)\left(e\in \mathbb{N}\right)$, i.e., $\underline{P}\left({ℒ}_{\text{e}}\right)\leq \underline{\zeta }\left({ℒ}_{\text{e}}\right)$ and $\bar{P}\left({ℒ}_{\text{e}}\right)\leq \bar{\zeta }\left({ℒ}_{\text{e}}\right)$. Then,
  (45) $$\begin{array}{c} HWA\left(P\left(L_{1}\right),P\left(L_{2}\right),\ldots ,P\left(L_{\text{n}}\right)\right)\leq HWA\left(\zeta \left(L_{1}\right),\zeta \left(L_{2}\right),\ldots ,\zeta \left(L_{\text{n}}\right)\right). \end{array}$$

**Proof**

Follow from Theorem 2.

### 4.2. *q*-Rung Orthopair Fuzzy Rough Geometric AInf

**Definition 14 .**

Consider that (*M*, *ζ*)∈*q*-ROF approximation space. Let $\zeta \left({ℒ}_{\text{e}}\right)=\left(\underline{\zeta }\left({ℒ}_{\text{e}}\right),\bar{\zeta }\left({ℒ}_{\text{e}}\right)\right)\in q-\text{ROFRS}\left(M\right)\left(e\in \mathbb{N}\right)$. Then, weighted geometric AInf is defined as follows:

(46) $$\begin{array}{c} WG\left(\zeta \left(L_{1}\right),\zeta \left(L_{2}\right),\ldots ,\zeta \left(L_{\text{n}}\right)\right)=\left(\overset{n}{\underset{e=1}{\prod }}{\left(\underline{\zeta }\left(L_{\text{e}}\right)\right)}^{\beta_{e}},\overset{n}{\underset{e=1}{\prod }}{\left(\bar{\zeta }\left(L_{\text{e}}\right)\right)}^{\beta_{e}}\right), \end{array}$$

where the weight of (*ζ*(*ℒ*_1_), *ζ*(*ℒ*_2_),…, *ζ*(*ℒ*_n_)) is (*β*_1_, *β*_2_,…*β*_*n*_)^*T*^, i.e., *β*_*e*_ ≥ 0; ∑_*e*=1_^*n*^*β*_*e*_=1.

**Theorem 7 .**

Consider (*M*, *ζ*)∈*q*-ROF AS. Let $\zeta \left({ℒ}_{\text{e}}\right)=\left(\underline{\zeta }\left({ℒ}_{\text{e}}\right),\bar{\zeta }\left({ℒ}_{\text{e}}\right)\right)\in q-\text{ROFRS}\left(M\right)\left(e\in \mathbb{N}\right)$ and the weight of (*ζ*(*ℒ*_1_), *ζ*(*ℒ*_2_),…, *ζ*(*ℒ*_n_)) be (*β*_1_, *β*_2_,…*β*_*n*_)^*T*^, i.e., *β*_*e*_ ≥ 0; ∑_*e*=1_^*n*^*β*_*e*_=1. Then, *WG* AInf is a transformation *D*^*n*^⟶*D*, i.e.,

(47) $$\begin{array}{c} WG\left(\zeta \left(L_{1}\right),\zeta \left(L_{2}\right),\ldots ,\zeta \left(L_{\text{n}}\right)\right)=\left(\overset{n}{\underset{e=1}{\prod }}{\left(\underline{\zeta }\left(L_{\text{e}}\right)\right)}^{\beta_{e}},\overset{n}{\underset{e=1}{\prod }}{\left(\bar{\zeta }\left(L_{\text{e}}\right)\right)}^{\beta_{e}}\right)\\ =\left\{\begin{array}{c} \left(t^{-1}\left(\sum_{e=1}^{n}\beta_{e}t\left(\underline{\mu_{e}}\right)\right),\sqrt[{q}]{s^{-1}\left(\sum_{e=1}^{n}\beta_{e}s\left({\underline{\nu_{e}}}^{q}\right)\right)}\right),\\ \left(t^{-1}\left(\sum_{e=1}^{n}\beta_{e}t\left(\bar{\mu_{e}}\right)\right),\sqrt[{q}]{s^{-1}\left(\sum_{e=1}^{n}\beta_{e}s\left({\bar{\nu_{e}}}^{q}\right)\right)}\right) \end{array}\right\}. \end{array}$$

For assigning values to *t* and *s* generators, we get Einstein operations for *q*-ROFRVs, similar to Einstein strict Archimedean norms.

(48) $$\begin{array}{c} WG^{\left(E\right)}\left(\zeta \left(L_{1}\right),\zeta \left(L_{2}\right),\ldots ,\zeta \left(L_{\text{n}}\right)\right)=\left(\overset{n}{\underset{e=1}{\prod }}{\left(\underline{\zeta }\left(L_{\text{e}}\right)\right)}^{\beta_{e}},\overset{n}{\underset{e=1}{\prod }}{\left(\bar{\zeta }\left(L_{\text{e}}\right)\right)}^{\beta_{e}}\right)\\ =\left\{\begin{array}{c} \left(\frac{\sqrt[{q}]{2\prod_{e=1}^{n}{\left({\underline{\mu_{e}}}^{q}\right)}^{\beta_{e}}}}{\sqrt[{q}]{\prod_{e=1}^{n}{\left(2-{\underline{\mu_{e}}}^{q}\right)}^{\beta_{e}}+\prod_{e=1}^{n}{\left({\underline{\mu_{e}}}^{q}\right)}^{\beta_{e}}}},\sqrt[{q}]{\frac{\prod_{e=1}^{n}{\left(1+{\underline{\nu_{e}}}^{q}\right)}^{\beta_{e}}\_\prod_{e=1}^{n}{\left(1-{\underline{\nu_{e}}}^{q}\right)}^{\beta_{e}}}{\prod_{e=1}^{n}{\left(1+{\underline{\nu_{e}}}^{q}\right)}^{\beta_{e}}+\prod_{e=1}^{n}{\left(1-{\underline{\nu_{e}}}^{q}\right)}^{\beta_{e}}}}\right),\\ \left(\frac{\sqrt[{q}]{2\overset{n}{\underset{e=1}{\prod }}{\left({\bar{\mu_{e}}}^{q}\right)}^{\beta_{e}}}}{\sqrt[{q}]{\overset{n}{\underset{e=1}{\prod }}{\left(2-{\bar{\mu_{e}}}^{q}\right)}^{\beta_{e}}+\overset{n}{\underset{e=1}{\prod }}{\left({\bar{\mu_{e}}}^{q}\right)}^{\beta_{e}}}},\sqrt[{q}]{\frac{\prod_{e=1}^{n}{\left(1+{\bar{\nu_{e}}}^{q}\right)}^{\beta_{e}}\_\prod_{e=1}^{n}{\left(1-{\bar{\nu_{e}}}^{q}\right)}^{\beta_{e}}}{\prod_{e=1}^{n}{\left(1+{\bar{\nu_{e}}}^{q}\right)}^{\beta_{e}}+\prod_{e=1}^{n}{\left(1-{\bar{\nu_{e}}}^{q}\right)}^{\beta_{e}}}}\right) \end{array}\right\}. \end{array}$$

**Proof**

The proof is similar to that of Theorem 1.

From the above analysis, $\zeta \left(ℒ\right)=\left(\underline{\zeta }\left(ℒ\right),\bar{\zeta }\left(ℒ\right)\right)$ is the *q*-ROFRV. So, by Definition 8, $\left(\prod_{e=1}^{n}{\left(\underline{\zeta }\left({ℒ}_{\text{e}}\right)\right)}^{\beta_{e}},\prod_{e=1}^{n}{\left(\bar{\zeta }\left({ℒ}_{\text{e}}\right)\right)}^{\beta_{e}}\right)$ are also *q*-ROFRVs. Therefore, *WG*(*ζ*(*ℒ*_1_), *ζ*(*ℒ*_2_),…, *ζ*(*ℒ*_n_)) is also a *q*-ROFRV under *q*-ROF AS (*M*, *ζ*).

Some important properties of the *q*-ROF rough weighted geometric operator are initiated in Theorem 8.

**Theorem 8 .**

Consider (*M*, *ζ*)∈*q*-ROF AS. Consider $\zeta \left({ℒ}_{\text{e}}\right)=\left(\underline{\zeta }\left({ℒ}_{\text{e}}\right),\bar{\zeta }\left({ℒ}_{\text{e}}\right)\right)\;\in \;q-\text{ROFRS}\left(M\right)\;\left(e\in \mathbb{N}\right)$ and (*β*_1_, *β*_2_,…*β*_*n*_)^*T*^ to be the weight of (*ζ*(*ℒ*_1_), *ζ*(*ℒ*_2_),…, *ζ*(*ℒ*_n_)), i.e., *β*_*e*_ ≥ 0; ∑_*e*=1_^*n*^*β*_*e*_=1. Then, some important properties of the *q*-ROF rough weighted geometric operator are described as follows:

(1) Idempotency: if $\zeta \left({ℒ}_{\text{e}}\right)=\zeta \left(ℒ\right)=\left(\underline{\zeta }\left(ℒ\right),\bar{\zeta }\left(ℒ\right)\right)$∀ *e* ∈ *ℕ*, then
  (49) $$\begin{array}{c} WG\left(\zeta \left(L_{1}\right),\zeta \left(L_{2}\right),\ldots ,\zeta \left(L_{\text{n}}\right)\right)=\zeta \left(L\right). \end{array}$$
(2) Boundedness: let ${\left(\zeta \left(ℒ\right)\right)}^{-}=\left(\underset{e}{\min}\underline{\zeta }\left({ℒ}_{\text{e}}\right),\underset{e}{\max}\bar{\zeta }\left({ℒ}_{\text{e}}\right)\right)$ and ${\left(\zeta \left(ℒ\right)\right)}^{+}=\left(\underset{e}{\max}\underline{\zeta }\left({ℒ}_{\text{e}}\right),\underset{e}{\min}\bar{\zeta }\left({ℒ}_{\text{e}}\right)\right)$. Then,
  (50) $$\begin{array}{c} {\left(\zeta \left(L\right)\right)}^{-}\leq WG\left(\zeta \left(L_{1}\right),\zeta \left(L_{2}\right),\ldots ,\zeta \left(L_{\text{n}}\right)\right)\leq {\left(\zeta \left(L\right)\right)}^{+}. \end{array}$$
(3) Monotonicity: let $P\left({ℒ}_{\text{e}}\right)=\left(\underline{P}\left({ℒ}_{\text{e}}\right),\bar{P}\left({ℒ}_{\text{e}}\right)\right)\;\in \;q-\text{ROFRS}\left(M\right)\;\left(e\in \mathbb{N}\right)$ such that $\underline{P}\left({ℒ}_{\text{e}}\right)\leq \underline{\zeta }\left({ℒ}_{\text{e}}\right)$ and $\bar{P}\left({ℒ}_{\text{e}}\right)\leq \bar{\zeta }\left({ℒ}_{\text{e}}\right)$. Then,
  (51) $$\begin{array}{c} WG\left(P\left(L_{1}\right),P\left(L_{2}\right),\ldots ,P\left(L_{\text{n}}\right)\right)\leq WG\left(\zeta \left(L_{1}\right),\zeta \left(L_{2}\right),\ldots ,\zeta \left(L_{\text{n}}\right)\right). \end{array}$$

**Proof**

Follow from Theorem 2.

**Definition 15 .**

Consider (*M*, *ζ*)∈*q*-ROF approximation space. Let $\zeta \left({ℒ}_{\text{e}}\right)=\left(\underline{\zeta }\left({ℒ}_{\text{e}}\right),\bar{\zeta }\left({ℒ}_{\text{e}}\right)\right)\in q-\text{ROFRS}\left(M\right)\left(e\in \mathbb{N}\right)$. Then, ordered weighted geometric AInf can be defined as in the following:

(52) $$\begin{array}{c} OWG\left(\zeta \left(L_{1}\right),\zeta \left(L_{2}\right),\ldots ,\zeta \left(L_{\text{n}}\right)\right)=\left(\overset{n}{\underset{e=1}{\prod }}{\left(\underline{\zeta }\left(L_{\xi \left(\text{e}\right)}\right)\right)}^{\beta_{e}},\overset{n}{\underset{e=1}{\prod }}{\left(\bar{\zeta }\left(L_{\xi \left(\text{e}\right)}\right)\right)}^{\beta_{e}}\right), \end{array}$$

where *ξ*(*e*) is denoted as the order according to (*ξ*(1), *ξ*(2), *ξ*(3),…, *ξ*(*n*)) and (*β*_1_, *β*_2_,…*β*_*n*_)^*T*^ and the weight of (*ζ*(*ℒ*_1_), *ζ*(*ℒ*_2_),…, *ζ*(*ℒ*_n_)) is (*β*_1_, *β*_2_,…*β*_*n*_)^*T*^, i.e., *β*_*e*_ ≥ 0; ∑_*e*=1_^*n*^*β*_*e*_=1.

**Theorem 9 .**

Consider that (*M*, *ζ*)∈*q*-ROF approximation space. Consider $\zeta \left({ℒ}_{\text{e}}\right)=\left(\underline{\zeta }\left({ℒ}_{\text{e}}\right),\bar{\zeta }\left({ℒ}_{\text{e}}\right)\right)\;\in \;q-\text{ROFRS}\left(M\right)$(*e* ∈ *ℕ*) and (*β*_1_, *β*_2_,…*β*_*n*_)^*T*^ to be the weight information of (*ζ*(*ℒ*_1_), *ζ*(*ℒ*_2_),…, *ζ*(*ℒ*_n_)) such that *β*_*e*_ ≥ 0; ∑_*e*=1_^*n*^*β*_*e*_=1. Then, the mapping of *OWG* AInf is *D*^*n*^⟶*D*, i.e.,

(53) $$\begin{array}{c} OWG\left(\zeta \left(L_{1}\right),\zeta \left(L_{2}\right),\ldots ,\zeta \left(L_{\text{n}}\right)\right)=\left(\overset{n}{\underset{e=1}{\prod }}{\left(\underline{\zeta }\left(L_{\xi \left(\text{e}\right)}\right)\right)}^{\beta_{e}},\overset{n}{\underset{e=1}{\prod }}{\left(\bar{\zeta }\left(L_{\xi \left(\text{e}\right)}\right)\right)}^{\beta_{e}}\right)\\ =\left\{\begin{array}{c} \left(t^{-1}\left(\sum_{e=1}^{n}\beta_{e}t\left(\underline{\mu_{\xi \left(e\right)}}\right)\right),\sqrt[{q}]{s^{-1}\left(\sum_{e=1}^{n}\beta_{e}s\left({\underline{\nu_{\xi \left(e\right)}}}^{q}\right)\right)}\right),\\ \left(t^{-1}\left(\sum_{e=1}^{n}\beta_{e}t\left(\bar{\mu_{\xi \left(e\right)}}\right)\right),\sqrt[{q}]{s^{-1}\left(\sum_{e=1}^{n}\beta_{e}s\left({\bar{\nu_{\xi \left(e\right)}}}^{q}\right)\right)}\right) \end{array}\right\}. \end{array}$$

For assigning values to *t* and *s* generators, we get Einstein operations for *q*-ROFRVs, similar to Einstein strict Archimedean norms.

(54) $$\begin{array}{c} OWG\left(\zeta \left(L_{1}\right),\zeta \left(L_{2}\right),\ldots ,\zeta \left(L_{\text{n}}\right)\right)=\left(\overset{n}{\underset{e=1}{\prod }}{\left(\underline{\zeta }\left(L_{\xi \left(\text{e}\right)}\right)\right)}^{\beta_{e}},\overset{n}{\underset{e=1}{\prod }}{\left(\bar{\zeta }\left(L_{\xi \left(\text{e}\right)}\right)\right)}^{\beta_{e}}\right)\\ =\left\{\begin{array}{c} \left(\sqrt[{q}]{\frac{\prod_{e=1}^{n}{\left(1+{\underline{\mu_{\xi \left(e\right)}}}^{q}\right)}^{\beta_{e}}\_\prod_{e=1}^{n}{\left(1-{\underline{\mu_{\xi \left(e\right)}}}^{q}\right)}^{\beta_{e}}}{\prod_{e=1}^{n}{\left(1+{\underline{\mu_{\xi \left(e\right)}}}^{q}\right)}^{\beta_{e}}+\overset{n}{\underset{e=1}{\prod }}\prod_{e=1}^{n}{\left(1-{\underline{\mu_{\xi \left(e\right)}}}^{q}\right)}^{\beta_{e}}}},\frac{\sqrt[{q}]{2\prod_{e=1}^{n}{\left({\left(\underline{\nu_{\xi \left(e\right)}}\right)}^{q}\right)}^{\beta_{e}}}}{\sqrt[{q}]{\prod_{e=1}^{n}{\left(2-{\underline{\nu_{\xi \left(e\right)}}}^{q}\right)}^{\beta_{e}}+\prod_{e=1}^{n}{\left({\left(\underline{\nu_{\xi \left(e\right)}}\right)}^{q}\right)}^{\beta_{e}}}}\right),\\ \left(\sqrt[{q}]{\frac{\prod_{e=1}^{n}{\left(1+{\bar{\mu_{\xi \left(e\right)}}}^{q}\right)}^{\beta_{e}}\_\prod_{e=1}^{n}{\left(1-{\bar{\mu_{\xi \left(e\right)}}}^{q}\right)}^{\beta_{e}}}{\prod_{e=1}^{n}{\left(1+{\bar{\mu_{\xi \left(e\right)}}}^{q}\right)}^{\beta_{e}}+\prod_{e=1}^{n}{\left(1-{\bar{\mu_{\xi \left(e\right)}}}^{q}\right)}^{\beta_{e}}}},\frac{\sqrt[{q}]{2\prod_{e=1}^{n}{\left({\left(\bar{\nu_{\xi \left(e\right)}}\right)}^{q}\right)}^{\beta_{e}}}}{\sqrt[{q}]{\prod_{e=1}^{n}{\left(2-{\bar{\nu_{\xi \left(e\right)}}}^{q}\right)}^{\beta_{e}}+\prod_{e=1}^{n}{\left({\left(\bar{\nu_{\xi \left(e\right)}}\right)}^{q}\right)}^{\beta_{e}}}}\right) \end{array}\right\}. \end{array}$$

**Proof**

Follow from Theorem 7.

**Theorem 10 .**

Consider (*M*, *ζ*)∈*q*-ROF approximation space. Let $\zeta \left({ℒ}_{\text{e}}\right)=\left(\underline{\zeta }\left({ℒ}_{\text{e}}\right),\bar{\zeta }\left({ℒ}_{\text{e}}\right)\right)\;\in \;q-\text{ROFRS}\left(M\right)\left(e\in \mathbb{N}\right)$ and (*β*_1_, *β*_2_,…*β*_*n*_)^*T*^ and the weight of (*ζ*(*ℒ*_1_), *ζ*(*ℒ*_2_),…, *ζ*(*ℒ*_n_)) be (*β*_1_, *β*_2_,…*β*_*n*_)^*T*^, i.e., *β*_*e*_ ≥ 0; ∑_*e*=1_^*n*^*β*_*e*_=1.

(1) Idempotency: if $\zeta \left({ℒ}_{\text{e}}\right)=\zeta \left(ℒ\right)=\left(\underline{\zeta }\left(ℒ\right),\bar{\zeta }\left(ℒ\right)\right)$∀ *e* ∈ *ℕ*, then
  (55) $$\begin{array}{c} OWG\left(\zeta \left(L_{1}\right),\zeta \left(L_{2}\right),\ldots ,\zeta \left(L_{\text{n}}\right)\right)=\zeta \left(L\right). \end{array}$$
(2) Boundedness: let ${\left(\zeta \left(ℒ\right)\right)}^{-}=\left(\underset{e}{\min}\underline{\zeta }\left({ℒ}_{\text{e}}\right),\underset{e}{\max}\bar{\zeta }\left({ℒ}_{\text{e}}\right)\right)$ and ${\left(\zeta \left(ℒ\right)\right)}^{+}=\left(\underset{e}{\max}\underline{\zeta }\left({ℒ}_{\text{e}}\right),\underset{e}{\min}\bar{\zeta }\left({ℒ}_{\text{e}}\right)\right)$. Then,
  (56) $$\begin{array}{c} {\left(\zeta \left(L\right)\right)}^{-}\leq OWG\left(\zeta \left(L_{1}\right),\zeta \left(L_{2}\right),\ldots ,\zeta \left(L_{\text{n}}\right)\right)\leq {\left(\zeta \left(L\right)\right)}^{+}. \end{array}$$
(3) Monotonicity: let $P\left({ℒ}_{\text{e}}\right)=\left(\underline{P}\left({ℒ}_{\text{e}}\right),\bar{P}\left({ℒ}_{\text{e}}\right)\right)\;\in \;q-\text{ROFRS}\left(M\right)\;\left(e\in \mathbb{N}\right)$ such that $\underline{P}\left({ℒ}_{\text{e}}\right)\leq \underline{\zeta }\left({ℒ}_{\text{e}}\right)$ and $\bar{P}\left({ℒ}_{\text{e}}\right)\leq \bar{\zeta }\left({ℒ}_{\text{e}}\right)$. Then,
  (57) $$\begin{array}{c} OWG\left(P\left(L_{1}\right),P\left(L_{2}\right),\ldots ,P\left(L_{\text{n}}\right)\right)\leq OWG\left(\zeta \left(L_{1}\right),\zeta \left(L_{2}\right),\ldots ,\zeta \left(L_{\text{n}}\right)\right). \end{array}$$

**Proof**

Follow from Theorem 2.

**Definition 16 .**

Consider (*M*, *ζ*)∈*q*-ROF AS. Let $\zeta \left({ℒ}_{\text{e}}\right)=\left(\underline{\zeta }\left({ℒ}_{\text{e}}\right),\bar{\zeta }\left({ℒ}_{\text{e}}\right)\right)\in q-\text{ROFRS}\left(M\right)\left(e\in \mathbb{N}\right)$. Then, hybrid weighted geometric AInf can be defined as in the following:

(58) $$\begin{array}{c} HWG\left(\zeta \left(L_{1}\right),\zeta \left(L_{2}\right),\ldots ,\zeta \left(L_{\text{n}}\right)\right)=\left(\overset{n}{\underset{e=1}{\prod }}{\left(\underline{\zeta }\left(L_{\xi \left(\text{e}\right)}^{\prime }\right)\right)}^{\eta_{e}},\overset{n}{\underset{e=1}{\prod }}{\left(\bar{\zeta }\left(L_{\xi \left(\text{e}\right)}^{\prime }\right)\right)}^{\eta_{e}}\right), \end{array}$$

where *ξ*(*e*) is represented as the order according to (*ξ*(1), *ξ*(2), *ξ*(3),…, *ξ*(*n*)) such that $\underline{\zeta }\left({ℒ}_{\xi \left(\text{e}\right)}^{\prime }\right)\left(\underline{\zeta }\left({ℒ}_{\xi \left(\text{e}\right)}^{\prime }\right)={\left(\underline{\zeta }\left({ℒ}_{\text{e}}\right)\right)}^{n\beta_{e}}:e\in \mathbb{N}\right)$ and $\bar{\zeta }\left({ℒ}_{\xi \left(\text{e}\right)}^{\prime }\right)\left(\bar{\zeta }\left({ℒ}_{\xi \left(\text{e}\right)}^{\prime }\right)={\left(\bar{\zeta }\left({ℒ}_{\text{e}}\right)\right)}^{n\beta_{e}}:e\in \mathbb{N}\right)$ and the weight of (*ζ*(*ℒ*_1_), *ζ*(*ℒ*_2_),…, *ζ*(*ℒ*_n_)) is (*β*_1_, *β*_2_,…*β*_*n*_)^*T*^, i.e., *β*_*e*_ ≥ 0; ∑_*e*=1_^*n*^*β*_*e*_=1. Also, (*η*_1_, *η*_2_,…*η*_*n*_)^*T*^ represent the associated weight of (*ζ*(*ℒ*_1_), *ζ*(*ℒ*_2_),…, *ζ*(*ℒ*_n_)), i.e., *η*_*e*_ ≥ 0; ∑_*e*=1_^*n*^*η*_*e*_=1.

**Theorem 11 .**

Consider (*M*, *ζ*)∈*q*-ROF AS. Let $\zeta \left({ℒ}_{\text{e}}\right)=\left(\underline{\zeta }\left({ℒ}_{\text{e}}\right),\bar{\zeta }\left({ℒ}_{\text{e}}\right)\right)\;\in \;q-\text{ROFRS}\left(M\right)\;\left(e\in \mathbb{N}\right)$ and the weight of (*ζ*(*ℒ*_1_), *ζ*(*ℒ*_2_),…, *ζ*(*ℒ*_n_)) be (*β*_1_, *β*_2_,…*β*_*n*_)^*T*^, i.e., *β*_*e*_ ≥ 0; ∑_*e*=1_^*n*^*β*_*e*_=1. Then, *HWG* AInf is a transformation *D*^*n*^⟶*D* with associated weight (*η*_1_, *η*_2_,…*η*_*n*_)^*T*^, i.e., *η*_*e*_ ≥ 0; ∑_*e*=1_^*n*^*η*_*e*_=1, i.e.,

(59) $$\begin{array}{c} HWG\left(\zeta \left(L_{1}\right),\zeta \left(L_{2}\right),\ldots ,\zeta \left(L_{\text{n}}\right)\right)=\left(\overset{n}{\underset{e=1}{\prod }}{\left(\underline{\zeta }\left(L_{\xi \left(\text{e}\right)}^{\prime }\right)\right)}^{\eta_{e}},\overset{n}{\underset{e=1}{\prod }}{\left(\bar{\zeta }\left(L_{\xi \left(\text{e}\right)}^{\prime }\right)\right)}^{\eta_{e}}\right)\\ =\left\{\begin{array}{c} \left(t^{-1}\left(\sum_{e=1}^{n}\eta_{e}t\left(\underline{\mu_{\xi \left(e\right)}^{\prime }}\right)\right),\sqrt[{q}]{s^{-1}\left(\sum_{e=1}^{n}\eta_{e}s\left({\underline{\nu_{\xi \left(e\right)}^{\prime }}}^{q}\right)\right)}\right),\\ \left(t^{-1}\left(\sum_{e=1}^{n}\eta_{e}t\left(\bar{\mu_{\xi \left(e\right)}^{\prime }}\right)\right),\sqrt[{q}]{s^{-1}\left(\sum_{e=1}^{n}\eta_{e}s\left({\bar{\nu_{\xi \left(e\right)}^{\prime }}}^{q}\right)\right)}\right) \end{array}\right\}. \end{array}$$

For assigning values to *t* and *s* generators, we get Einstein operations for *q*-ROFRVs, similar to Einstein strict Archimedean norms.

(60) $$\begin{array}{c} HWG\left(\zeta \left(L_{1}\right),\zeta \left(L_{2}\right),\ldots ,\zeta \left(L_{\text{n}}\right)\right)=\left(\overset{n}{\underset{e=1}{\prod }}{\left(\underline{\zeta }\left(L_{\xi \left(\text{e}\right)}^{\prime }\right)\right)}^{\eta_{e}},\overset{n}{\underset{e=1}{\prod }}{\left(\bar{\zeta }\left(L_{\xi \left(\text{e}\right)}^{\prime }\right)\right)}^{\eta_{e}}\right)\\ =\left\{\begin{array}{c} \left(\frac{\sqrt[{q}]{2\prod_{e=1}^{n}{\left({\underline{\mu_{\xi \left(e\right)}^{\prime }}}^{q}\right)}^{\eta_{e}}}}{\sqrt[{q}]{\prod_{e=1}^{n}{\left(2-{\underline{\mu_{\xi \left(e\right)}^{\prime }}}^{q}\right)}^{\eta_{e}}+\prod_{e=1}^{n}{\left({\underline{\mu_{\xi \left(e\right)}^{\prime }}}^{q}\right)}^{\eta_{e}}}},\sqrt[{q}]{\frac{\prod_{e=1}^{n}{\left(1+{\underline{\nu_{\xi \left(e\right)}^{\prime }}}^{q}\right)}^{\eta_{e}}\_\prod_{e=1}^{n}{\left(1-{\underline{\nu_{\xi \left(e\right)}^{\prime }}}^{q}\right)}^{\eta_{e}}}{\prod_{e=1}^{n}{\left(1+{\underline{\nu_{\xi \left(e\right)}^{\prime }}}^{q}\right)}^{\eta_{e}}+\prod_{e=1}^{n}{\left(1-{\underline{\nu_{\xi \left(e\right)}^{\prime }}}^{q}\right)}^{\eta_{e}}}}\right),\\ \left(\frac{\sqrt[{q}]{2\prod_{e=1}^{n}{\left({\bar{\mu_{\xi \left(e\right)}^{\prime }}}^{q}\right)}^{\eta_{e}}}}{\sqrt[{q}]{\prod_{e=1}^{n}{\left(2-{\underline{\mu_{\xi \left(e\right)}^{\prime }}}^{q}\right)}^{\eta_{e}}+\prod_{e=1}^{n}{\left({\bar{\mu_{\xi \left(e\right)}^{\prime }}}^{q}\right)}^{\eta_{e}}}},\sqrt{\frac{\prod_{e=1}^{n}{\left(1+{\bar{\nu_{\xi \left(e\right)}^{\prime }}}^{q}\right)}^{\eta_{e}}\_\prod_{e=1}^{n}{\left(1-{\bar{\nu_{\xi \left(e\right)}^{\prime }}}^{q}\right)}^{\eta_{e}}}{\prod_{e=1}^{n}{\left(1+{\bar{\nu_{\xi \left(e\right)}^{\prime }}}^{q}\right)}^{\eta_{e}}+\prod_{e=1}^{n}{\left(1-{\bar{\nu_{\xi \left(e\right)}^{\prime }}}^{q}\right)}^{\eta_{e}}}}\right) \end{array}\right\}. \end{array}$$

**Proof**

Follow from Theorem 7.

**Theorem 12 .**

Consider (*M*, *ζ*)∈*q*-ROF approximation space. Let $\zeta \left({ℒ}_{\text{e}}\right)=\left(\underline{\zeta }\left({ℒ}_{\text{e}}\right),\bar{\zeta }\left({ℒ}_{\text{e}}\right)\right)\;\in \;q-\text{ROFRS}\left(M\right)\left(e\in \mathbb{N}\right)$ and (*β*_1_, *β*_2_,…*β*_*n*_)^*T*^ be the weight of (*ζ*(*ℒ*_1_), *ζ*(*ℒ*_2_),…, *ζ*(*ℒ*_n_)), i.e., *β*_*e*_ ≥ 0; ∑_*e*=1_^*n*^*β*_*e*_=1. Then, some important properties of the *q*-ROF rough hybrid weighted geometric operator are described as follows:

(1) Idempotency: if $\zeta \left({ℒ}_{\text{e}}\right)=\zeta \left(ℒ\right)=\left(\underline{\zeta }\left(ℒ\right),\bar{\zeta }\left(ℒ\right)\right)$∀ *e* ∈ *ℕ*, then
  (61) $$\begin{array}{c} HWG\left(\zeta \left(L_{1}\right),\zeta \left(L_{2}\right),\ldots ,\zeta \left(L_{\text{n}}\right)\right)=\zeta \left(L\right). \end{array}$$
(2) Boundedness: let ${\left(\zeta \left(ℒ\right)\right)}^{-}=\left(\underset{e}{\min}\underline{\zeta }\left({ℒ}_{\text{e}}\right),\underset{e}{\max}\bar{\zeta }\left({ℒ}_{\text{e}}\right)\right)$ and ${\left(\zeta \left(ℒ\right)\right)}^{+}=\left(\underset{e}{\max}\underline{\zeta }\left({ℒ}_{\text{e}}\right),\underset{e}{\min}\bar{\zeta }\left({ℒ}_{\text{e}}\right)\right)$. Then,
  (62) $$\begin{array}{c} {\left(\zeta \left(L\right)\right)}^{-}\leq HWG\left(\zeta \left(L_{1}\right),\zeta \left(L_{2}\right),\ldots ,\zeta \left(L_{\text{n}}\right)\right)\leq {\left(\zeta \left(L\right)\right)}^{+}. \end{array}$$
(3) Monotonicity: let $P\left({ℒ}_{\text{e}}\right)=\left(\underline{P}\left({ℒ}_{\text{e}}\right),\bar{P}\left({ℒ}_{\text{e}}\right)\right)\;\in \;q-\text{ROFRS}\left(M\right)\;\left(e\in \mathbb{N}\right)$ such that $\underline{P}\left({ℒ}_{\text{e}}\right)\leq \underline{\zeta }\left({ℒ}_{\text{e}}\right)$ and $\bar{P}\left({ℒ}_{\text{e}}\right)\leq \bar{\zeta }\left({ℒ}_{\text{e}}\right)$. Then,
  (63) $$\begin{array}{c} HWG\left(P\left(L_{1}\right),P\left(L_{2}\right),\ldots ,P\left(L_{\text{n}}\right)\right)\leq HWG\left(\zeta \left(L_{1}\right),\zeta \left(L_{2}\right),\ldots ,\zeta \left(L_{\text{n}}\right)\right). \end{array}$$

**Proof**

Follow from Theorem 2.

## 5. EDAS Methodology Based on *q*-Rung Orthopair Fuzzy Einstein Rough Aggregation Operators

We present a methodology for dealing with uncertainties in decision-making (DM) while dealing with *q*-ROFR information. Suppose a DM problem with a set of *m* alternatives {ℷ_1_, ℷ_2_,…, ℷ_*e*_} and {*ℒ*_1_, *ℒ*_2_,…., *ℒ*_h_} denote a set of attributes with (*β*_1_, *β*_2_,….. , *β*_*h*_)^*T*^ being the weights, i.e., *β*_*t*_ ∈ [0,1], ∑_*t*=1_^*h*^*β*_*t*_=1. Allow a group of decision makers (DMs) $\left\{{\overset{{}^{\circ}}{D}}_{1},{\overset{{}^{\circ}}{D}}_{2},\ldots ,{\overset{{}^{\circ}}{D}}_{\hat{\chi }}\right\}$ to examine the reliability of the *k*th alternative ℷ_*k*_ under the *t*th attribute *ℒ*_t_, and ${\left(\eta_{1},\eta_{2},\ldots ,\eta_{\hat{\chi }}\right)}^{T}$ are DM weights such that *η*_*s*_ ∈ [0,1], $\sum_{s=1}^{\hat{\chi }}\eta_{s}=1$. The expert evaluation matrix is described as follows:

(64) $$\begin{array}{c} \text{M}={\left[\zeta \left(L_{ij}^{\hat{j}}\right)\right]}_{m\times n}\\ =\left[\begin{array}{cccc} \left(\underline{\zeta }\left(L_{11}\right),\bar{\zeta }\left(L_{11}\right)\right) & \left(\underline{\zeta }\left(L_{12}\right),\bar{\zeta }\left(L_{12}\right)\right) & \cdots & \left(\underline{\zeta }\left(L_{1\text{j}}\right),\bar{\zeta }\left(L_{1\text{j}}\right)\right)\\ \left(\underline{\zeta }\left(L_{21}\right),\bar{\zeta }\left(L_{21}\right)\right) & \left(\underline{\zeta }\left(L_{22}\right),\bar{\zeta }\left(L_{22}\right)\right) & \cdots & \left(\underline{\zeta }\left(L_{2\text{j}}\right),\bar{\zeta }\left(L_{2\text{j}}\right)\right)\\ \left(\underline{\zeta }\left(L_{31}\right),\bar{\zeta }\left(L_{31}\right)\right) & \left(\underline{\zeta }\left(L_{32}\right),\bar{\zeta }\left(L_{32}\right)\right) & \cdots & \left(\underline{\zeta }\left(L_{3\text{j}}\right),\bar{\zeta }\left(L_{3\text{j}}\right)\right)\\ \vdots & \vdots & \ddots & \vdots \\ \left(\underline{\zeta }\left(L_{\text{i}1}\right),\bar{\zeta }\left(L_{\text{i}1}\right)\right) & \left(\underline{\zeta }\left(L_{\text{i}2}\right),\bar{\zeta }\left(L_{\text{i}2}\right)\right) & \cdots & \left(\underline{\zeta }\left(L_{\text{ij}}\right),\bar{\zeta }\left(L_{\text{ij}}\right)\right) \end{array}\right], \end{array}$$

where $\underline{\zeta }\left({ℒ}_{\text{ij}}\right)=\left\{\left(℘,\mu_{\underline{\zeta }\left({ℒ}_{\text{ij}}\right)}\left(℘\right),\nu_{\underline{\zeta }\left({ℒ}_{\text{ij}}\right)}\left(℘\right)\right):℘\in M\right\}$ and $\bar{\zeta }\left({ℒ}_{\text{ij}}\right)=\left\{\left(℘,\mu_{\bar{\zeta }\left({ℒ}_{\text{ij}}\right)}\left(℘\right),\nu_{\bar{\zeta }\left({ℒ}_{\text{ij}}\right)}\left(℘\right)\right):℘\in M\right\}$ such that $0\leq {\left(\mu_{\underline{\zeta }\left({ℒ}_{\text{ij}}\right)}\left(℘\right)\right)}^{q}+{\left(\nu_{\underline{\zeta }\left({ℒ}_{\text{ij}}\right)}\left(℘\right)\right)}^{q}\leq 1$ and $0\leq {\left(\mu_{\bar{\zeta }\left({ℒ}_{\text{ij}}\right)}\left(℘\right)\right)}^{q}+{\left(\nu_{\bar{\zeta }\left({ℒ}_{\text{ij}}\right)}\left(℘\right)\right)}^{q}\leq 1$ are the *q*-ROF rough values.

 Step 1: construct the experts' evaluation matrices ${\left(E\right)}^{\hat{\chi }}$.
  (65) $$\begin{array}{c} \left[\begin{array}{cccc} \left(\underline{\zeta }\left(L_{11}\right),\bar{\zeta }\left(L_{11}\right)\right) & \left(\underline{\zeta }\left(L_{12}\right),\bar{\zeta }\left(L_{12}\right)\right) & \cdots & \left(\underline{\zeta }\left(L_{1\text{j}}\right),\bar{\zeta }\left(L_{1\text{j}}\right)\right)\\ \left(\underline{\zeta }\left(L_{21}\right),\bar{\zeta }\left(L_{21}\right)\right) & \left(\underline{\zeta }\left(L_{22}\right),\bar{\zeta }\left(L_{22}\right)\right) & \cdots & \left(\underline{\zeta }\left(L_{2\text{j}}\right),\bar{\zeta }\left(L_{2\text{j}}\right)\right)\\ \left(\underline{\zeta }\left(L_{31}\right),\bar{\zeta }\left(L_{31}\right)\right) & \left(\underline{\zeta }\left(L_{32}\right),\bar{\zeta }\left(L_{32}\right)\right) & \cdots & \left(\underline{\zeta }\left(L_{3\text{j}}\right),\bar{\zeta }\left(L_{3\text{j}}\right)\right)\\ \vdots & \vdots & \ddots & \vdots \\ \left(\underline{\zeta }\left(L_{\text{i}1}\right),\bar{\zeta }\left(L_{\text{i}1}\right)\right) & \left(\underline{\zeta }\left(L_{\text{i}2}\right),\bar{\zeta }\left(L_{\text{i}2}\right)\right) & \cdots & \left(\underline{\zeta }\left(L_{\text{ij}}\right),\bar{\zeta }\left(L_{\text{ij}}\right)\right) \end{array}\right], \end{array}$$
 where the number of experts is represented by $\hat{\chi }$.
 Step 2: evaluate normalized experts' matrices ${\left(N\right)}^{\hat{\chi }}$, that is,
  (66) $$\begin{array}{c} {\left(N\right)}^{\hat{\chi }}=\left\{\begin{array}{cc} \zeta \left(L_{\text{ij}}\right)=\left(\underline{\zeta }\left(L_{\text{ij}}\right),\bar{\zeta }\left(L_{\text{ij}}\right)\right)=\left(\left(\underline{\mu_{ij}},\underline{\nu_{ij}}\right),\left(\bar{\mu_{ij}},\bar{\nu_{ij}}\right)\right) & \text{if for benefit,}\\ {\left(\zeta \left(L_{\text{ij}}\right)\right)}^{c}=\left({\left(\underline{\zeta }\left(L_{\text{ij}}\right)\right)}^{c},{\left(\bar{\zeta }\left(L_{\text{ij}}\right)\right)}^{c}\right)=\left(\left(\underline{\nu_{ij}},\underline{\mu_{ij}}\right),\left(\bar{\nu_{ij}},\bar{\mu_{ij}}\right)\right) & \text{if for cost.} \end{array}\right. \end{array}$$
 Step 3: evaluate the collective expert information based on the *q*-ROF Einstein rough weighted averaging operator.
  (67) $$\begin{array}{c} WA^{\left(E\right)}\left(\zeta \left(L_{1}\right),\zeta \left(L_{2}\right),\ldots ,\zeta \left(L_{\text{n}}\right)\right)=\left(\sum_{e=1}^{n}\beta_{e}\underline{\zeta }\left(L_{\text{e}}\right),\sum_{e=1}^{n}\beta_{e}\bar{\zeta }\left(L_{\text{e}}\right)\right)\\ =\left\{\begin{array}{c} \left(\frac{\sqrt[{q}]{2\prod_{e=1}^{n}{\left({\underline{\mu_{e}}}^{q}\right)}^{\beta_{e}}}}{\sqrt[{q}]{\prod_{e=1}^{n}{\left(2-{\underline{\mu_{e}}}^{q}\right)}^{\beta_{e}}+\prod_{e=1}^{n}{\left({\underline{\mu_{e}}}^{q}\right)}^{\beta_{e}}}},\sqrt[{q}]{\frac{\prod_{e=1}^{n}{\left(1+{\underline{\nu_{e}}}^{q}\right)}^{\beta_{e}}\_\prod_{e=1}^{n}{\left(1-{\underline{\nu_{e}}}^{q}\right)}^{\beta_{e}}}{\prod_{e=1}^{n}{\left(1+{\underline{\nu_{e}}}^{q}\right)}^{\beta_{e}}+\prod_{e=1}^{n}{\left(1-{\underline{\nu_{e}}}^{q}\right)}^{\beta_{e}}}}\right),\\ \left(\frac{\sqrt[{q}]{2\overset{n}{\underset{e=1}{\prod }}{\left({\bar{\mu_{e}}}^{q}\right)}^{\beta_{e}}}}{\sqrt[{q}]{\overset{n}{\underset{e=1}{\prod }}{\left(2-{\bar{\mu_{e}}}^{q}\right)}^{\beta_{e}}+\overset{n}{\underset{e=1}{\prod }}{\left({\bar{\mu_{e}}}^{q}\right)}^{\beta_{e}}}},\sqrt[{q}]{\frac{\prod_{e=1}^{n}{\left(1+{\bar{\nu_{e}}}^{q}\right)}^{\beta_{e}}\_\prod_{e=1}^{n}{\left(1-{\bar{\nu_{e}}}^{q}\right)}^{\beta_{e}}}{\prod_{e=1}^{n}{\left(1+{\bar{\nu_{e}}}^{q}\right)}^{\beta_{e}}+\prod_{e=1}^{n}{\left(1-{\bar{\nu_{e}}}^{q}\right)}^{\beta_{e}}}}\right) \end{array}\right\}. \end{array}$$
 Step 4: evaluate the value of the AVS by using suggested aggregation operators for considering the alternative w.r.t the attribute.
  (68) $$\begin{array}{c} AVS={\left[AVS_{j}\right]}_{1\times n}={\left[\frac{1}{m}\sum_{i=1}^{m}\zeta \left(L_{\text{ij}}^{\text{n}}\right)\right]}_{1\times n}\\ =\left\{\begin{array}{c} \left(\sqrt[{q}]{\frac{\prod_{i=1}^{m}{\left(1+{\underline{\mu_{ij}}}^{q}\right)}^{1/m}\_\prod_{i=1}^{m}{\left(1-{\underline{\mu_{ij}}}^{q}\right)}^{1/m}}{\prod_{i=1}^{m}{\left(1+{\underline{\mu_{ij}}}^{q}\right)}^{1/m}+\prod_{i=1}^{m}{\left(1-{\underline{\mu_{ij}}}^{q}\right)}^{1/m}}},\frac{\sqrt[{q}]{2\prod_{i=1}^{m}{\left({\underline{\nu_{ij}}}^{q}\right)}^{1/m}}}{\sqrt[{q}]{\overset{m}{\underset{i=1}{\prod }}{\left(2-{\underline{\nu_{ij}}}^{q}\right)}^{1/m}+\overset{m}{\underset{i=1}{\prod }}{\left({\underline{\nu_{ij}}}^{q}\right)}^{1/m}}}\right),\\ \left(\sqrt[{q}]{\frac{\prod_{i=1}^{m}{\left(1+{\bar{\mu_{ij}}}^{q}\right)}^{1/m}\_\prod_{i=1}^{m}{\left(1-{\bar{\mu_{ij}}}^{q}\right)}^{1/m}}{\prod_{i=1}^{m}{\left(1+{\bar{\mu_{ij}}}^{q}\right)}^{1/m}+\prod_{i=1}^{m}{\left(1-{\bar{\mu_{ij}}}^{q}\right)}^{1/m}}},\frac{\sqrt[{q}]{2\prod_{i=1}^{m}{\left({\bar{\nu_{ij}}}^{q}\right)}^{1/m}}}{\sqrt[{q}]{\prod_{i=1}^{m}{\left(2-{\bar{\nu_{ij}}}^{q}\right)}^{1/m}+\prod_{i=1}^{m}{\left({\bar{\nu_{ij}}}^{q}\right)}^{1/m}}}\right) \end{array}\right\}. \end{array}$$
 Step 5: utilizing the value of the AVS, evaluate the values of the PDAS and NDAS as follows:
  (69) $$\begin{array}{c} PDAS_{ij}={\left[PDAS_{ij}\right]}_{m\times n}\\ =\frac{\max\left(0,\left[So\left(\zeta \left(L_{ij}^{n}\right)\right)-So\left(AVS_{j}\right)\right]\right)}{So\left(AVS_{j}\right)}. \end{array}$$
  (70) $$\begin{array}{c} N\;DA\;S_{ij}={\left[N\;DA\;S_{ij}\right]}_{m\times n}\\ \;=\frac{\max\left(0,\left[So\left(AVS_{j}\right)-So\left(\zeta \left(L_{\text{ij}}^{\text{n}}\right)\right)\right]\right)}{So\left(AVS_{j}\right)}. \end{array}$$
 Step 6: evaluate the positive *Sp*_*i*_ and negative *Sn*_*i*_ weighted distance as follows:
  (71) $$\begin{array}{c} Sp_{i}=\sum_{j=1}^{n}\beta_{j}P\;DA\;S_{ij}, \end{array}$$
  (72) $$\begin{array}{c} Sn_{i}=\sum_{j=1}^{n}\beta_{j}N\;DA\;S_{ij}. \end{array}$$
 Step 7: now, evaluate normalized positive *Sp*_*i*_ and negative *Sn*_*i*_ weighted distances as
  (73) $$\begin{array}{c} NSp_{i}=\frac{Sp_{i}}{\max_{i}\left(Sp_{i}\right)}, \end{array}$$
  (74) $$\begin{array}{c} NSn_{i}=1-\frac{Sn_{i}}{\max_{i}\left(Sn_{i}\right)}. \end{array}$$
 Step 8: utilizing the value of *NSp*_*i*_ and *NSn*_*i*_, appraisal score *ASo*_*i*_ can be calculated as follows:
  (75) $$\begin{array}{c} ASo_{i}=\frac{1}{2}\left(NSp_{i}+NSn_{i}\right). \end{array}$$
 Step 9: rate the alternatives and select the higher *ASo*_*i*_ value.

Figure 1 shows the graphical framework of the proposed method.

## 6. Numerical Application of the Proposed Algorithm

Throughout this part, a practical MAGDM problem involving determining an acceptable mode of farming among various types of agrifarming is used to ensure that the established approach is applicable and feasible.

### 6.1. Real-Life Case Study: Robotic Agrifarming

Green agriculture refers to the application of sustainable development concepts to agriculture, such as ensuring the food production and fibers while maintaining the economic and social constraints that ensure the production's long-term viability. Sustainable farming, for example, decreases the use of pesticides, which can be dangerous to farmers' and consumers' health. Precision agriculture and smart farming are major elements of sustainable agriculture. Growing crops and raising livestock are the job or business of farming. Farming includes raising animals and growing crops, both of which provide us with food and raw materials. Farming started nearly 5,000 years ago, but the precise date and origin are unknown. Farming is a way of life, not just a career. Really, we are all farmers, and we all enjoy farming, whether at home or in the fields. This love of gardening must be a lifelong habit, whether you are young or old. Food prices will skyrocket as a result of this land destruction, and we will have to pay even more for our everyday food needs. To get out of this situation, farmers must concentrate on growing yield production through the use of agricultural robots. The use of robots in agriculture is an example of creativity that goes beyond invention. Agricultural farming acts as an industry, and in the new era, it will develop into a high-tech industry. “Agribots” or “agri-robots” are other terms for agricultural robots [41]. Four key alternatives are linked to sustainable agriculture:

1. Good crop production (ℷ_1_): develop productive, self-sufficient, and cost-effective production systems that earn well. Another advantage is that farming gives us a decent income as well as jobs, food, and services to the majority of people who are currently poor. Furthermore, it enables the development of rural areas and the establishment of social connections between the rural and urban worlds.
2. Environmental protection (ℷ_2_): manage the quality of air, water, and soil while preserving and protecting biodiversity and territories. Agriculture's first benefit is environmental protection as it reduces deforestation and natural resource depletion, increases biodiversity, and reduces carbon emissions.
3. Natural resources' availability (ℷ_3_): improve the quality in which natural resources are used. Another key difficulty that green agriculture faces is the rapid degradation and loss of natural resources. The availability of natural resources improves farming and benefits us.
4. Food security and productivity (ℷ_4_): increase food production and distribution energy efficiency. With the world's population increasing and persistently high levels of hunger and poverty, sustainable agriculture yields must solve the problem of food security by generating more in less time.

In addition, the four alternatives are assessed using five criteria. The attributes of robotic agrifarming are given as follows:

1. High quality production (*ℒ*_1_): certain farming factors, such as soil and time of ripeness, have an effect on the quality of the products. On wheat, barley, rice, and other cereals, maturity level and degree of dryness matter.
2. Limiting the need for manual labor (*ℒ*_2_): since the labor cost in agriculture, i.e., farming, is so high, qualified employees and manual labor are in high demand.
3. Decreasing the cost of production (*ℒ*_3_): in the field of agriculture, there is an interesting idea for decreasing production costs which includes the use of robots. We must deal with certain uncontrollable variables such as environmental conditions, buying various brands of seeds, and using a huge number of chemicals.
4. Completion of a time-consuming project (*ℒ*_4_): the use of automation, according to scientists, technologists, scholars, and farmers, will solve the complicated project in a quick and easy manner.
5. Consistent role to complete a project (*ℒ*_5_): to maintain a consistent location, the farm must be managed using artificial intelligence from seeding to harvesting.

The invited decision makers are composed of three experts.

(76) $$\begin{array}{c} \text{Experts}=\left\{{\left(E\right)}^{1},{\left(E\right)}^{2},{\left(E\right)}^{3}\right\}, \end{array}$$

for which every expert panel must offer unified assessment *q*-ROFR data with unknown expert and criteria weight details..

 Step 1: Tables2–4 contain *q*-ROF rough value expert evaluation information.
 Step 2: Tables 5–7 represent normalized expert information.
 Step 3: collected information in the form of *q*-ROF rough information is given in Table 8.
 Step 4: AVS values based on the proposed *q*-ROF Einstein rough aggregation operators are given in Tables 9 and 10.
 Step 5: *P*  *DA*  *S*_*ij*_ and *N*  *DA*  *S*_*ij*_ are calculated as follows.
     Case 1: for the Einstein WA aggregation operator (given in Tables 11 and 12).
     Case 2: for the Einstein OWA aggregation operator (given in Tables 13 and 14).
     Case 3: for the Einstein HWA aggregation operator (given in Tables 15 and 16).
     Case 4: for the Einstein WG aggregation operator (given in Tables 17 and 18).
     Case 5: for the Einstein OWG aggregation operator (given in Tables 19 and 20).
     Case 6: for the Einstein HWG aggregation operator (given in Tables 21 and 22).
 Step 6: the positive *Sp*_*i*_ and negative *Sn*_*i*_ weighted distance based on proposed operators are given in Tables 23 and 24.
 Step 7: normalized positive *Sp*_*i*_ and negative *Sn*_*i*_ weighted distances based on proposed operators are given in Tables 25 and 26.
 Step 8: appraisal score of collective preference alternative values is listed in Table 27.
 Step 9: alternatives' ranking ℷ_*k*_(*k*=1,2,…., 4) is listed in Table 28.

We obtained that alternative ℷ_2_ is the best among the alternatives based on the above computational process, and thus, it is strongly suggested.

## 7. Conclusion

In this manuscript, we have presented a new FS extension called *q*-ROFRS. This concept will provide a more versatile and efficient basis for fuzzy system modeling and decision-making under uncertainties due to the implementation of the concept of the rough set (RS) theory. Based on the developed concept, a list of aggregation operators such as *q*-ROFR weighted averaging and geometric operators are established based on algebraic and Einstein norms. Furthermore, the basic desirable characteristics of developed operators are discussed in detail. Moreover, the concept of the entropy and distance measures is presented to determine the decision makers' unknown weights as well as attributes' weight information. Furthermore, we have successfully applied the proposed approach to a MADMP involving the selection of the best agrifarming robots in agriculture. In contrast to some current methods, numerical results indicate that the *q*-ROFRS-based method is more realistic and versatile in real-world applications. To demonstrate the feasibility and superiority of the proposed methods, a comparative review of the final ranking and optimal decision in robotic agrifarming calculated by the suggested methods with some previous methods is given. We will expand this work in the future to Frank aggregation operators and Hamacher operators to solve a variety of real-world problems and make decisions under uncertainties in different fields such as computational intelligence and medical diagnosis.

## Figures and Tables

**Figure 1:** Graphical framework of the proposed method.

**Table 1:** *q*-ROF relation from set *M* to *M*.

*ζ*	*℘*_1_	*℘*_2_	*℘*_3_	*℘*_4_
*℘*_1_	(0.93, 0.11)	(0.72, 0.14)	(0.76, 0.34)	(0.57, 0.06)
*℘*_2_	(0.77, 0.31)	(0.85, 0.26)	(0.47,0.43)	(0.85, 0.13)
*℘*_3_	(0.47, 0.66)	(0.67, 0.19)	(0.91, 0.06)	(0.60, 0.30)
*℘*_4_	(0.86, 0.12)	(0.46, 0.08)	(0.72, 0.22)	(0.79, 0.14)

**Table 2:** Expert information (*E*)^1^.

	£_1_	£_2_	£_3_	£_4_	£_5_
ℷ_1_	((0.3, 0.6), (0.2, 0.8))	((0.1, 0.8), (0.2, 0.7))	((0.1, 0.9), (0.3, 0.4))	((0.1, 0.9), (0.2, 0.7))	((0.1, 0.5), (0.2, 0.4))
ℷ_2_	((0.2, 0.5), (0.1, 0.9))	((0.2, 0.6), (0.3, 0.4))	((0.1, 0.4), (0.1, 0.8))	((0.2, 0.7), (0.1, 0.5))	((0.1, 0.4), (0.4, 0.6))
ℷ_3_	((0.4, 0.6), (0.3, 0.5))	((0.3, 0.6), (0.2, 0.5))	((0.1, 0.6), (0.3, 0.4))	((0.5, 0.4), (0.6, 0.3))	((0.4, 0.6), (0.3, 0.4))
ℷ_4_	((0.1, 0.7), (0.2, 0.4))	((0.6, 0.4), (0.4, 0.5))	((0.1, 0.2), (0.2, 0.5))	((0.4, 0.5), (0.5, 0.3))	((0.3, 0.5), (0.2, 0.4))

**Table 3:** Expert information (*E*)^2^.

	£_1_	£_2_	£_3_	£_4_	£_5_
ℷ_1_	((0.1;0.6), (0.2;0.3))	((0.2; 0.8), (0.3; 0.6))	((0.3; 0.6), (0.1; 0.7))	((0.1; 0.5), (0.3; 0.7))	((0.1; 0.9), (0.1; 0.8))
ℷ_2_	((0.1;0.4), (0.3;0.5))	((0.1; 0.9), (0.2; 0.4))	((0.5; 0.4), (0.1; 0.4))	((0.3; 0.4), (0.7; 0.2))	((0.2; 0.8), (0.5; 0.4))
ℷ_3_	((0.2;0.7), (0.7;0.2))	((0.2; 0.4), (0.6; 0.2))	((0.3; 0.5), (0.3; 0.5))	((0.7; 0.2), (0.2; 0.7))	((0.3; 0.5), (0.1; 0.3))
ℷ_4_	((0.5;0.5), (0.2;0.6))	((0.3; 0.6), (0.3; 0.4))	((0.1; 0.3), (0.4; 0.5))	((0.2; 0.6), (0.5; 0.4))	((0.3; 0.6), (0.3; 0.2))

**Table 4:** Expert information (*E*)^3^.

	£_1_	£_2_	£_3_	£_4_	£_5_
ℷ_1_	((0.1;0.7), (0.1;0.2))	((0.2; 0.8), (0.3; 0.6))	((0.3; 0.7), (0.2; 0.6))	((0.2; 0.5), (0.1; 0.4))	((0.1; 0.8), (0.2; 0.7))
ℷ_2_	((0.2;0.7), (0.4;0.3))	((0.3; 0.5), (0.3; 0.4))	((0.1; 0.5), (0.6; 0.3))	((0.3; 0.7), (0.1; 0.5))	((0.3; 0.6), (0.1; 0.4))
ℷ_3_	((0.2;0.4), (0.1;0.5))	((0.1; 0.9), (0.1; 0.9))	((0.3; 0.4), (0.6; 0.2))	((0.2; 0.8), (0.4; 0.3))	((0.4; 0.6), (0.2; 0.3))
ℷ_4_	((0.1;0.5), (0.3;0.7))	((0.2; 0.5), (0.6; 0.4))	((0.2; 0.3), (0.3; 0.1))	((0.1; 0.3), (0.2; 0.4))	((0.2; 0.4), (0.3; 0.5))

**Table 5:** Normalized expert information (*N*)^1^.

	£_1_	£_2_	£_3_	£_4_	£_5_
ℷ_1_	((0.6;0.3), (0.8;0.2))	((0.8; 0.1), (0.7; 0.2))	((0.9; 0.1), (0.4; 0.3))	((0.9; 0.1), (0.7; 0.2))	(0.5; 0.1), (0.4; 0.2))
ℷ_2_	((0.5;0.2), (0.9;0.1))	((0.6; 0.2), (0.4; 0.3))	((0.4; 0.1), (0.8; 0.1))	((0.7; 0.2), (0.5; 0.1))	((0.4; 0.1), (0.6; 0.4))
ℷ_3_	((0.6;0.4), (0.5;0.3))	((0.6; 0.3), (0.5; 0.2))	((0.6; 0.1), (0.4; 0.3))	((0.4; 0.5), (0.3; 0.6))	((0.6; 0.4), (0.4; 0.3))
ℷ_4_	((0.7;0.1), (0.4;0.2))	((0.4; 0.6), (0.5; 0.4))	((0.2; 0.1), (0.5; 0.2))	((0.5; 0.4), (0.3; 0.5))	((0.5; 0.3), (0.4; 0.2))

**Table 6:** Normalized expert information (*N*)^2^.

	£_1_	£_2_	£_3_	£_4_	£_5_
ℷ_1_	((0.6;0.1), (0.3;0.2))	((0.8; 0.2), (0.6; 0.3))	((0.6; 0.3), (0.7; 0.1))	((0.5; 0.1), (0.7; 0.3))	((0.9; 0.1), (0.8; 0.1))
ℷ_2_	((0.4;0.1), (0.5;0.3))	((0.9; 0.1), (0.4; 0.2))	((0.4; 0.5), (0.4; 0.1))	((0.4; 0.3), (0.2; 0.7))	((0.8; 0.2), (0.4; 0.5))
ℷ_3_	((0.7;0.2), (0.2;0.7))	((0.4; 0.2), (0.2; 0.6))	((0.5; 0.3), (0.5; 0.3))	((0.2; 0.7), (0.7; 0.2))	((0.5; 0.3), (0.3; 0.1))
ℷ_4_	((0.5;0.5), (0.6;0.2))	((0.6; 0.3), (0.4; 0.3))	((0.3; 0.1), (0.5; 0.4))	((0.6; 0.2), (0.4; 0.5))	((0.6; 0.3), (0.2; 0.3))

**Table 7:** Normalized expert information (*N*)^3^.

	£_1_	£_2_	£_3_	£_4_	£_5_
ℷ_1_	((0.7;0.1), (0.2;0.1))	((0.8; 0.2), (0.6; 0.3))	((0.7; 0.3), (0.6; 0.2))	((0.5; 0.2), (0.4; 0.1))	((0.8; 0.1), (0.7; 0.2))
ℷ_2_	((0.7;0.2), (0.3;0.4))	((0.5; 0.3), (0.4; 0.3))	((0.5; 0.1), (0.3; 0.6))	((0.7; 0.3), (0.5; 0.1))	((0.6; 0.3), (0.4; 0)
ℷ_3_	((0.4;0.2), (0.5;0.1))	((0.9; 0.1), (0.9; 0.1))	((0.4; 0.3), (0.2; 0.6))	((0.8; 0.2), (0.3; 0.4))	((0.6; 0.4), (0.3; 0.2))
ℷ_4_	((0.5;0.1), (0.7;0.3))	((0.5; 0.2), (0.4; 0.6))	((0.3; 0.2), (0.1; 0.3))	((0.3; 0.1), (0.4; 0.2))	((0.4; 0.2), (0.5; 0.3))

**Table 8:** Collected expert's information.

	£_1_	£_2_	£_3_	£_4_	£_5_
ℷ_1_	((0.64;0.13), (0.46;0.15))	((0.8; 0.16), (0.63; 0.26))	((0.75; 0.22), (0.58; 0.18))	((0.67; 0.13), (0.60; 0.17))	((0.78; 0.1), (0.67; 0.15))
ℷ_2_	((0.55;0.15), (0.62;0.24))	((0.71; 0.18), (0.4; 0.26))	((0.43; 0.17), (0.51; 0.20))	((0.61; 0.26), (0.40; 0.20))	((0.63; 0.19), (0.46; 0.26))
ℷ_3_	((0.57;0.24), (0.40;0.27))	((0.71; 0.17), (0.65; 0.23))	((0.49; 0.22), (0.36; 0.39))	((0.54; 0.40), (0.45; 0.36))	((0.56; 0.36), (0.32; 0.18))
ℷ_4_	((0.56;0.17), (0.59;0.23))	((0.50; 0.32), (0.43; 0.42))	((0.27; 0.13), (0.36; 0.29))	((0.46; 0.19), (0.37; 0.36))	((0.49; 0.25), (0.37; 0.26))

**Table 9:** AVS (averaging aggregation operators).

	*WA*	*OWA*	*HWA*
£_1_	((0.584; 0.176), (0.526; 0.224))	((0.668; 0.149), (0.636; 0.215))	((0.614; 0.185), (0.553; 0.235))
£_2_	((0.698; 0.204), (0.539; 0.290))	((0.662; 0.210), (0.462; 0.268))	((0.863; 0.246), (0.656; 0.349))
£_3_	((0.515; 0.183), (0.463; 0.259))	((0.591; 0.206), (0.448; 0.236))	((0.577; 0.202), (0.512; 0.285))
£_4_	((0.580; 0.231), (0.465; 0.264))	((0.515; 0.183), (0.463; 0.259))	((0.432; 0.173), (0.347; 0.198))
£_5_	((0.636; 0.208), (0.473; 0.213))	((0.579; 0.267), (0.439; 0.268))	((0.568; 0.187), (0.423; 0.191))

**Table 10:** AVS (geometric aggregation operators).

	*WG*	*OWG*	*HWG*
£_1_	((0.567; 0.208), (0.446; 0.271))	((0.610; 0.176), (0.548; 0.251))	((0.0122; 0.0002), (0.0036; 0.0006))
£_2_	((0.640; 0.234), (0.481; 0.329))	((0.621; 0.253), (0.416; 0.252))	((0.0250; 0.0344), (0.0060; 0.0015))
£_3_	((0.458; 0.217), (0.398; 0.313))	((0.571; 0.234), (0.436; 0.330))	((0.0040; 0.0001), (0.0021; 0.0011))
£_4_	((0.513; 0.284), (0.426; 0.336))	((0.543; 0.255), (0.422; 0.357))	((0.0052; 0.0010), (0.0020; 0.0009))
£_5_	((0.593; 0.237), (0.430; 0.242))	((0.429; 0.261), (0.370; 0.299))	((0.0129; 0.0003), (0.0025; 0.0002))

**Table 11:** *PDAS*_*ij*_ (Einstein WA operator).

	£_1_	£_2_	£_3_	£_4_	
ℷ_1_	(0.3596)	(0.0939)	(0.1596)	(0.1644)	(0.1904)
ℷ_2_	(0.0218)	(0.0001)	(0.0149)	(0.0025)	(0.0001)
ℷ_3_	(0.0001)	(0.0819)	(0.0001)	(0.0001)	(0.0001)
ℷ_4_	(0.0139)	(0.0001)	(0.0001)	(0.0001)	(0.0001)

**Table 12:** *NDAS*_*ij*_ (Einstein WA operator).

	£_1_	£_2_	£_3_	£_4_	
ℷ_1_	(0.0001)	(0.0001)	(0.0001)	(0.0001)	(0.0001)
ℷ_2_	(0.0001)	(0.0286)	(0.0001)	(0.0001)	(0.0171)
ℷ_3_	(0.9375)	(0.0001)	(0.1158)	(0.1274)	(0.1242)
ℷ_4_	(0.0001)	(0.2022)	(0.1294)	(0.1029)	(0.1243)

**Table 13:** *PDAS*_*ij*_ (Einstein OWA operator).

	£_1_	£_2_	£_3_	£_4_	
ℷ_1_	(0.0881)	(0.1338)	(0.1431)	(0.1596)	(0.1307)
ℷ_2_	(0.0001)	(0.0067)	(0.017)	(0.015)	(0.0293)
ℷ_3_	(0.0090)	(0.0001)	(0.0001)	(0.0001)	(0.0001)
ℷ_4_	(0.0001)	(0.0001)	(0.0001)	(0.0001)	(0.0001)

**Table 14:** *NDAS*_*ij*_ (Einstein OWA operator).

	£_1_	£_2_	£_3_	£_4_	
ℷ_1_	(0.0001)	(0.0001)	(0.0001)	(0.0001)	(0.0001)
ℷ_2_	(0.0580)	(0.0001)	(0.0001)	(0.0001)	(0.0001)
ℷ_3_	(0.0001)	(0.0716)	(0.0938)	(0.1158)	(0.1041)
ℷ_4_	(0.0654)	(0.1105)	(0.1194)	(0.1294)	(0.1190)

**Table 15:** *PDAS*_*ij*_ (Einstein HWA operator).

	£_1_	£_2_	£_3_	£_4_	
ℷ_1_	(0.0368)	(0.0938)	(0.1661)	(0.1318)	(0.1787)
ℷ_2_	(0.0223)	(0.0000)	(0.0110)	(0.0032)	(0.0001)
ℷ_3_	(0.0001)	(0.0803)	(0.0001)	(0.0001)	(0.0001)
ℷ_4_	(0.0140)	(0.0001)	(0.0001)	(0.0001)	(0.0001)

**Table 16:** *NDAS*_*ij*_ (Einstein HWA operator).

	£_1_	£_2_	£_3_	£_4_	
ℷ_1_	(0.0001)	(0.0001)	(0.0001)	(0.0001)	(0.0001)
ℷ_2_	(0.0001)	(0.0440)	(0.0001)	(0.0001)	(0.0134)
ℷ_3_	(0.0974)	(0.0001)	(0.1291)	(0.0998)	(0.1126)
ℷ_4_	(0.0001)	(0.2393)	(0.1437)	(0.0804)	(0.1127)

**Table 17:** *PDAS*_*ij*_ (Einstein WG operator).

	£_1_	£_2_	£_3_	£_4_	
ℷ_1_	(0.0545)	(0.1669)	(0.2239)	(0.2254)	(0.2196)
ℷ_2_	(0.0215)	(0.0071)	(0.0014)	(0.0152)	(0.0001)
ℷ_3_	(0.0001)	(0.0218)	(0.0001)	(0.0001)	(0.0001)
ℷ_4_	(0.0428)	(0.0001)	(0.0001)	(0.0001)	(0.0001)

**Table 18:** *NDAS*_*ij*_ (Einstein WG operator).

	£_1_	£_2_	£_3_	£_4_	
ℷ_1_	(0.0001)	(0.0001)	(0.0001)	(0.0001)	(0.0001)
ℷ_2_	(0.0001)	(0.0001)	(0.0001)	(0.0001)	(0.0139)
ℷ_3_	(0.1038)	(0.0001)	(0.0744)	(0.1563)	(0.0849)
ℷ_4_	(0.0001)	(0.1746)	(0.0941)	(0.0548)	(0.0926)

**Table 19:** *PDAS*_*ij*_ (Einstein OWG operator).

	£_1_	£_2_	£_3_	£_4_	
ℷ_1_	(0.1357)	(0.1793)	(0.1655)	(0.2086)	(0.1936)
ℷ_2_	(0.0001)	(0.0178)	(0.0269)	(0.0013)	(0.0401)
ℷ_3_	(0.0001)	(0.0001)	(0.0001)	(0.0001)	(0.0001)
ℷ_4_	(0.0001)	(0.0001)	(0.0001)	(0.0001)	(0.0001)

**Table 20:** *NDAS*_*ij*_ (Einstein OWG operator).

	£_1_	£_2_	£_3_	£_4_	
ℷ_1_	(0.0001)	(0.0001)	(0.0001)	(0.0001)	(0.0001)
ℷ_2_	(0.0521)	(0.0001)	(0.0001)	(0.0001)	(0.0001)
ℷ_3_	(0.0429)	(0.0806)	(0.0701)	(0.0848)	(0.1259)
ℷ_4_	(0.0323)	(0.0883)	(0.1022)	(0.1023)	(0.0591)

**Table 21:** *PDAS*_*ij*_ (Einstein HWG operator).

	£_1_	£_2_	£_3_	£_4_	
ℷ_1_	(0.0040)	(0.0533)	(0.0252)	(0.0079)	(0.0210)
ℷ_2_	(0.0003)	(0.0174)	(0.0001)	(0.0027)	(0.0006)
ℷ_3_	(0.0001)	(0.0172)	(0.0001)	(0.0001)	(0.0006)
ℷ_4_	(0.0041)	(0.0048)	(0.0001)	(0.0001)	(0.0001)

**Table 22:** *NDAS*_*ij*_ (Einstein HWG operator).

	£_1_	£_2_	£_3_	£_4_	
ℷ_1_	(0.0001)	(0.0001)	(0.0001)	(0.0001)	(0.0001)
ℷ_2_	(0.0001)	(0.0001)	(0.0001)	(0.0001)	(0.0001)
ℷ_3_	(0.0006)	(0.0026)	(0.0001)	(0.0033)	(0.0024)
ℷ_4_	(0.0001)	(0.0001)	(0.0001)	(0.00161)	(0.0046)

**Table 23:** Result of *S*_*pi*_ (*i* = 1, 2, 3, and 4).

	*S*_*p1*_	*S*_*p2*_	*S*_*p3*_	*S*_*p4*_
WA	0.1241	0.0082	0.0196	0.0029
OWA	0.1296	0.0129	0.0019	0.0001
HWA	0.1187	0.0076	0.0192	0.0029
WG	0.1741	0.0088	0.0052	0.0090
OWG	0.1740	0.0176	0.0001	0.0001
HWG	0.0242	0.0047	0.0042	0.0020

**Table 24:** Result of *S*_*ni*_ (*i* = 1, 2, 3, and 4).

	*S*_*n1*_	*S*_*n2*_	*S*_*n3*_	*S*_*n4*_
WA	0.0001	0.0099	0.0866	0.1148
OWA	0.0001	0.0121	0.0739	0.1073
HWA	0.0001	0.0130	0.0841	0.1214
WG	0.0001	0.0025	0.0769	0.0875
OWG	0.0001	0.0109	0.0791	0.0764
HWG	0.0001	0.0001	0.0016	0.0010

**Table 25:** Result of normalized *S*_*pi*_ (*i* = 1, 2, 3, and 4).

	*NS*_*p1*_	*NS*_*p2*_	*NS*_*p3*_	*NS*_*p4*_
WA	1.0000	0.0666	0.1583	0.0235
OWA	1.0000	0.0995	0.0147	0.0000
HWA	1.0000	0.0641	0.1623	0.0248
WG	1.0000	0.0508	0.0300	0.0517
OWG	1.0000	0.1013	0.0000	0.0000
HWG	1.0000	0.1978	0.1762	0.0836

**Table 26:** Result of normalized *S*_*ni*_ (*i* = 1, 2, 3, and 4).

	*NS*_*n1*_	*NS*_*n2*_	*NS*_*n3*_	*NS*_*n4*_
WA	0.9999	0.9130	0.2453	0.0001
OWA	0.9999	0.8864	0.3112	0.0001
HWA	0.9999	0.8928	0.3069	0.0001
WG	0.9999	0.9713	0.1209	0.0001
OWG	0.9999	0.8618	0.0001	0.0343
HWG	0.9999	0.9999	0.0001	0.3493

**Table 27:** Appraisal score values.

Operators	*So*(ℷ_1_)	*So*(ℷ_2_)	*So*(ℷ_3_)	*So*(ℷ_4_)
WA	0.999	0.489	0.201	0.011
OWA	0.999	0.492	0.162	0.001
HWA	0.999	0.478	0.234	0.012
WG	0.999	0.510	0.075	0.025
OWG	0.999	0.481	0.001	0.017
HWG	0.999	0.598	0.088	0.205

**Table 28:** Ranking of the alternatives.

Operators	Score	Top
WA	*So*(ℷ_1_) > *So*(ℷ_2_) > *So*(ℷ_3_) > *So*(ℷ_4_)	ℷ_1_
OWA	*So*(ℷ_1_) > *So*(ℷ_2_) > *So*(ℷ_3_) > *So*(ℷ_4_)	ℷ_1_
HWA	*So*(ℷ_1_) > *So*(ℷ_2_) > *So*(ℷ_3_) > *So*(ℷ_4_)	ℷ_1_
WG	*So*(ℷ_1_) > *So*(ℷ_2_) > *So*(ℷ_3_) > *So*(ℷ_4_)	ℷ_1_
OWG	*So*(ℷ_1_) > *So*(ℷ_2_) > *So*(ℷ_4_) > *So*(ℷ_3_)	ℷ_1_
HWG	*So*(ℷ_1_) > *So*(ℷ_2_) > *So*(ℷ_4_) > *So*(ℷ_3_)	ℷ_1_

## Data Availability

The data used in this manuscript are hypothetical and can be used by anyone by just citing this article.
